The article "Appraisal and Simulation on Codynamics of Pneumonia and Meningitis with Vaccination Intervention: From a Mathematical Model Perspective" was published in 2022. Journal: Comput Math Methods Med.

# Appraisal and Simulation on Codynamics of Pneumonia and Meningitis with Vaccination Intervention: From a Mathematical Model Perspective

**DOI:** 10.1155/2022/9945047

**Published:** 2022-11-28

**Authors:** Belela Samuel Kotola, Dawit Melese Gebru, Haileyesus Tessema Alemneh

**Affiliations:** ^1^Department of Mathematics, Debre Berhan University, Debre Berhan, Ethiopia; ^2^Departments of Mathematics, Oda Bultum University, Chiro, Ethiopia; ^3^Department of Mathematics, Bahir Dar University, Bahir Dar, Ethiopia; ^4^Department of Mathematics, University of Gondar, Gondar, Ethiopia

## Abstract

The membranes that encompass the brain and spinal cord become inflamed by the potentially fatal infectious disease called pneumococcal meningitis. Pneumonia and meningitis “coinfection” refers to the presence of both conditions in a single host. In this work, we accounted for the dynamics of pneumonia and meningitis coinfection in communities by erroneously using a compartment model to analyze and suggest management techniques to stakeholders. We have used the next generation matrix approach and derived the effective reproduction numbers. When the reproduction number is less than one, the constructed model yields a locally asymptotically stable disease-free equilibrium point. Additionally, we conducted a sensitivity analysis to determine how different factors affected the incidence and transmission rate, which revealed that both the pneumonia and meningitis transmission rates are extremely sensitive. The performance of our numerical simulation demonstrates that the endemic equilibrium point of the pneumonia and meningitis coinfection model is locally asymptotically stable when max{ *ℛ*_1_, *ℛ*_2_} > 1. Finally, as preventative and control measures for the coinfection of pneumonia and meningitis illness, the stakeholders must concentrate on reducing the transmission rates, reducing vaccination wane rates, and boosting the portion of vaccination rates for both pneumonia and meningitis.

## 1. Introduction

The word “epidemiology” is derived from the Greek term “demos,” which means “people,” and “logos,” which means “the study of”. In other words, the term “epidemiology” has its roots in the study of the experiences of a population. Despite the fact that many definitions have been provided, the one that best encapsulates the fundamental ideas and public health perspective of epidemiology is: “Epidemiology is the study of the prevalence and causes of health-related conditions or incidents in particular populations, as well as the application of this information to the prevention or treatment of health issues” [1, 2]. In epidemiology, the frequency and distribution of health events in a population are studied.

The article "Appraisal and Simulation on Codynamics of Pneumonia and Meningitis with Vaccination Intervention: From a Mathematical Model Perspective" was published in 2022. Journal: Comput Math Methods Med.

By the term “frequency,” we not only mean the number of health events, such as the number of cases of meningitis or diabetes in a population, but also the correlation between that number and the size of the population [2, 3].

The underlying premise of epidemiology is that disease does not develop in a community at random but rather develops only when an individual has the proper confluence of risk factors or determinants. Individuals are the “patients” of clinicians, whereas communities are the “patients” of epidemiologists. In light of this, while dealing with a patient who is unwell, the clinician and the epidemiologist have separate duties. When a patient with diarrheal illness first shows up, for instance, both parties are concerned with making the right diagnosis [3–5].

A potentially fatal infection called pneumococcal meningitis inflames the membranes that cover the brain and spinal cord. The meninges, which are these layers, serve to shield the brain from damage and infection [5]. Millions of people have died as a result of pneumonia, an airborne disease that is caused by breathing harmful organisms, primarily *Streptococcus pneumonia*. Other illnesses, including meningitis, ear infections, and sinus infections, are also brought on by these bacteria [5–7]. Moreover, these illnesses can afflict people of all ages, from infants to the elderly. Pneumonia is particularly hazardous when the immune system is weakened, as in infants or the elderly, or when it is concomitant with another illness like meningitis [7, 8]. Pneumonia is a common coinfection that occurs at the time of admission in cases of bacterial meningitis and is independently linked to a poor prognosis and death [9].

The most frequent pneumococcal infection in children are caused by 13 different varieties of pneumococcal bacteria. There are vaccines named PCV13, which can protect against these types, and PPSV23, which can protect against 23 other types. For the sake of this investigation, we have studied prior work by other researchers who used mathematical modeling to explain the transmission and spread of coinfections with pneumonia and meningitis, such as [7, 10–13]. The majority of these investigations were carried out to identify community-level infectious disease control methods. To our knowledge, no one has created and examined the three kinds of vaccine independently in a mathematical model of meningitis and pneumonia coinfection in a specific community. As a result, this recently proposed study considers the dynamics of meningitis and pneumonia in communities, utilizing a deterministic compartmental model to analyze and recommend appropriate management techniques to actors. Therefore, we are driven and intrigued to investigate the three vaccine kinds for meningitis and pneumonia coinfection in this work by developing a mathematical model of meningitis and pneumonia coinfection combined with regulating techniques. We have laid up the basic framework for this investigation as follows: in Section 2, we outline and develop the compartmental mathematical model of coinfection with meningitis and pneumonia. The model analysis includes the equilibrium points, fundamental reproduction numbers, and stability analysis of the submodels and the main model also presented in Section 2. Numerical simulations and sensitivity analysis are presented in Section 3. The study's discussion and conclusion were then finalized.

The article "Appraisal and Simulation on Codynamics of Pneumonia and Meningitis with Vaccination Intervention: From a Mathematical Model Perspective" was published in 2022. Journal: Comput Math Methods Med.

## 2. Mathematical Model Formulations and Its Qualitative Analysis

In this section we have proposed a mathematical model which depend upon the assumption and present the qualitative properties of the constructed model.

### 2.1. Baseline Model Formulation and Assumptions

We have developed the new model by expanding the model which was developed previously by another researcher based on the following hypotheses. Under this study, we consider homogenous population and that the factors such as sex, social status, and race do not affect the probability of being infected. The model subdivides the human total population *N*(*t*) into nine mutually-exclusive compartments, namely, susceptible population *S*(*t*), pneumonia-only infectious *P*_*I*_(t), meningitis-only infectious  *M*_*I*_(t), meningitis and pneumonia coinfectious *MP*_*I*_(t), treated class  *T*(*t*), meningitis vaccinated M_*V*_(t), pneumonia vaccinated  P_*V*_(t), class of people who take both vaccines of pneumonia and meningitis (PCV13 Pneumococcal conjugate vaccine) group  *MP*_*V*_(*t*), and recovered class (R). The recovery from natural immunity and the effects of vertical transmission to pneumonia and meningitis were assumed to be insignificant in this study. Epidemiologically, individuals in the removed/recovered compartment *R*(*t*) do not attain permanent immunity so that we are assigned such case by the parameter *Y*.

In this study the mass action-incidence rate of new infections are used, and the modification parameters *ω*_1_ and  *ω*_2_ are the factors that describe the fact of how infectiousness level of pneumonia increases the susceptibility level to meningitis disease and vice versa, respectively. The meningitis disease is assumed to be transmitted after effective contact between the susceptible and meningitis infectious classes with effective contact rate *a*, where *a* is a composite parameter that measures the meningitis contact rate  *κ* and the probability of transmission upon contact  *q*. Additionally, pneumonia disease is assumed to be transmitted after effective contact between the susceptible and pneumonia infectious classes with effective contact rate  *b*, where *b* is a composite parameter which measure the pneumonia infectious contact rate *c* and the probability of transmission upon contact *p*. Individuals can get meningitis by contact rate *a* from a meningitis-only infected or coinfected person with force of infection of meningitis *α*_1_ = *a*(*M*_*I*_ + *ℯ*_1_*MP*_*I*_)  and join *M*_*I*_ compartment where *ℯ*_1_ is the modification parameter.

The article "Appraisal and Simulation on Codynamics of Pneumonia and Meningitis with Vaccination Intervention: From a Mathematical Model Perspective" was published in 2022. Journal: Comput Math Methods Med.

An individual can get pneumonia with contact rate of *b* from a pneumonia-only infected or coinfected person with force of infection of pneumonia  *α*_2_ = *b*(*P*_*I*_ + *ℯ*_2_*MP*_*I*_) and join the  *P*_*I*_ compartment with modification parameter *ℯ*_2_. Pneumonia-only infected individuals also can get an additional meningitis infection with force of infection and modification parameter  *ω*_1_*α*_1_ and join coinfected compartment  *MP*_*I*_. The coinfected compartment increases because of individuals that come from meningitis-only infected compartment are infected by pneumonia with force of infection and modification parameter  *ω*_2_ *α*_2_. Since the coinfected individuals are aware of the disease, they remain there in the treated compartment even if they are free from either pneumonia or meningitis until they are free from all the diseases. The parameters used in the model are described in Table 1.

Using the above assumptions and parameters, we have constructed the following schematic diagram that is given in Figure 1.

From the diagram given in Figure 1, the corresponding dynamical systems will be as follows from the assumptions of the model and using the above basic model assumption we have the following flow chart.

(1) $$\begin{array}{c} \left.\begin{array}{c} \frac{dS}{dt}=\left(1-\pi \right)\lambda +\phi \;P_{V}+\varphi M_{V}+YR–\left(\alpha_{1}+\alpha_{2}+\mu \right)S,\\ \frac{dM_{V}}{dt}=\left(1-\rho \right)\pi \lambda -\left(\mu +\varphi +\varepsilon_{1}\right)M_{V},\\ \frac{dP_{V}}{dt}=\rho \pi \lambda -\left(\mu +\phi +\varepsilon_{2}\right)P_{V},\\ \frac{d{MP}_{V}}{dt}=\varepsilon_{1}M_{V}+\varepsilon_{2}P_{V}-\mu {MP}_{V},\\ \frac{dM_{I}}{dt}=\alpha_{1}S–\left(\;\omega_{2}\alpha_{2}+\tau_{1}+\delta_{1}+\mu \right)M_{I},\\ \frac{dP_{I}}{dt}=\alpha_{2}S-\left(\;\omega_{1}\alpha_{1}+\tau_{2}+\delta_{2}+\mu \right)P_{I},\\ \frac{d{MP}_{I}}{dt}=\omega_{1}\alpha_{1}P_{I}+\omega_{2}\alpha_{2}M_{I}-\left(\tau_{3}+\delta_{3}+\mu \right){MP}_{I},\\ \frac{d\text{T}}{dt}=\tau_{1}M_{I}+\tau_{2}P_{I}+\tau_{3}{MP}_{I}-\left(\beta +\mu \right)\text{T},\\ \frac{d\text{R}}{dt}=\beta T-\left(Y+\mu \right)R. \end{array}\right\} \end{array}$$

This system of differential equation is the mathematical representation of full meningitis and pneumonia model which is the combination of the two diseases. In the next section, we have studied the qualitative behavior of the constructed model. For simplification of our work, we split the full meningitis-pneumonia coinfection model into submodels, which are meningitis-only and pneumonia-only models. First, we will study the qualitative behavior of the submodel and then qualitative behavior of the full model is followed.

The article "Appraisal and Simulation on Codynamics of Pneumonia and Meningitis with Vaccination Intervention: From a Mathematical Model Perspective" was published in 2022. Journal: Comput Math Methods Med.

### 2.2. Positivity of Solutions and Invariant Region of the Only Pneumonia-Infected Model

In this subsection, we have considered the model of pneumonia only in the absence of meningitis disease. This procedure will help us to summarize and conclude some properties of the full coinfected model depending on the properties of sub models. To gate this submodel from the full model, we set, *M*_*I*_ = *MP*_*I*_ = 0, and we have the following dynamical system.

The corresponding dynamical systems are as follow.

(2) $$\begin{array}{c} \left.\begin{array}{c} \frac{dS}{dt}=\left(1-\pi \right)\lambda +\phi \;P_{V}+YR–\left(\alpha_{2}+\mu \right)S,\\ \frac{dP_{I}}{dt}=\alpha_{2}S-\left(\tau_{2}+\delta_{2}+\mu \right)P_{I},\\ \frac{dP_{V}}{dt}=\pi \lambda -\left(\mu +\phi \right)P_{V},\\ \frac{d\text{T}}{dt}=\tau_{2}P_{I}-\left(\beta +\mu \right)\text{T},\\ \frac{d\text{R}}{dt}=\beta T-\left(Y+\mu \right)R. \end{array}\right\} \end{array}$$

For the dynamical systems to be epidemiologically meaningful as well as well-posed, we need to prove that all the state variables of dynamical systems are nonnegative.

**Theorem 1 .**

All the populations of the system with positive initial conditions are positive.

Proof: assume *S*(0) > 0, *P*_*I*_(0) > 0, *P*_*V*_(0) > 0, *T*(0) > 0 and *R*(0) > 0 are positive for time *t* > 0 and for all nonnegative parameters.

First, let us take *T* = sup{*t* > 0 such that S (*t*′) > 0, *P*_*I*_(*t*′) > 0, *P*_*V*_(*t*′) > 0, *T*(*t*′) > 0  and  *R*(*t*′) > 0, *t*′ ∈ [0, *t*]}.

From the first equation of system (2), we do have *dS*/*dt* = (1 − *π*)*λ* + *ϕ* *P*_*V*_ + *YR*–(*α*_2_ + *μ*)*S*⇒*S*(*t*) = *S*(0)*e*^−∫_0_^*T*^(*α*_2_ + *μ*)*dt*′^ + *e*^−∫_0_^*T*^(*α*_2_ + *μ*)*dt*′^[∫_0_^*T*^*e*^∫_0_^*T*^(*α*_2_ + *μ*)*dt*′^[(1 − *π*)*λ* + *YR* + *ϕ* *P*_*V*_]*dt*] > 0⇒*S*(*t*) > 0.

There, *S*(*t*) is positive. Following the same procedure, all the remaining state variables are nonnegative. Therefore, from proof, we can conclude that whenever the initial values of the systems are all nonnegative, then all the solutions of our dynamical system are positive.

The article "Appraisal and Simulation on Codynamics of Pneumonia and Meningitis with Vaccination Intervention: From a Mathematical Model Perspective" was published in 2022. Journal: Comput Math Methods Med.

**Theorem 2 .**

The total human population of the dynamical system (2) is positively closed in the closed invariant set *Ω*_1_ = {(*S*, *P*_*I*,_ *P*_*V*,_*T*, *R*)*ϵ*ℝ_+_^4^ : *N*_1_ ≤ (*λ*/*μ*)}.

Furthermore, the system's nonnegative solutions are all constrained, and it may exhibit the persistence property under any nonnegative initial concentration conditions [14].

Proof: assume the total population of the model is  *N*_1_. To get an invariant region, which shows boundedness of solution, it can be obtained as follows.

(3) $$\begin{array}{c} \;N_{1}=S+P_{I}+P_{V}+T+R\Rightarrow \frac{dN_{1}}{dt}=\lambda -\mu S-\delta_{2}P_{I}-\mu P_{I}-\mu P_{V}-\mu \text{T}-\mu R, \end{array}$$

(4) $$\begin{array}{c} \frac{\text{d}{\text{N}}_{1}}{\text{dt}}=\lambda -\mu {\text{N}}_{1}-\delta_{2}{\text{P}}_{\text{I}}\Rightarrow \frac{\text{d}{\text{N}}_{1}}{\text{dt}}+\mu {\text{N}}_{1}\leq \lambda , \end{array}$$

(5) $$\begin{array}{c} N_{1}\left(t\right)\leq N_{0}e^{-\mu t}+\frac{\lambda }{\mu }\Rightarrow \underset{t⟶\infty }{\lim}N_{1}\left(t\right)\leq \frac{\lambda }{\mu }, \end{array}$$

⇒0 ≤ *N*_1_ ≤ *λ*/*μ* .

Therefore, the dynamical system that we do have is bounded.

### 2.3. Existence and Stability of Disease-Free Equilibrium Point

The disease-free equilibrium point is obtained by making all the equations equal to zero, provided that  *P*_*I*_ = 0  and the obtained disease-free equilibrium point is given by

(6) $$\begin{array}{c} E_{p}^{0}=\left(S^{O},{P_{V,}}^{O}\;{P_{I}}^{O},T^{0},R^{O}\;\right)=\left(\frac{\lambda }{\mu }\left[\frac{\left(1-\pi \right)\left(\mu +\phi \right)+\pi \phi }{\left(\mu +\phi \right)}\right],\frac{\pi \lambda }{\left(\mu +\phi \right)},0,0,0\right). \end{array}$$

#### 2.3.1. Effective Reproduction Number

The reproduction number is the number of secondary cases produced by one infectious individual joining in a completely susceptible population during its infectious period [15–17].

Using the next generation matrix method, we have obtained the effective reproduction number of pneumonia-infected-only submodel, which is  *ℛ*_*ef*(*p*)_ = (*λb*/*μ*)((1 − *π*)(*μ* + *ϕ*) + *πϕ*/(*μ* + *ϕ*)(*τ*_2_ + *δ*_2_ + *μ*)).

**Theorem 3 .**

The disease-free equilibrium point *E*_*p*_^0^ of the model in system (2) is locally asymptotically stable if the effective reproduction number *ℛ*_*ef*(*p*)_ < 1 and is unstable if  *ℛ*_*ef*(*p*)_ > 1.

Proof: from the Jacobean matrix  *J*(*E*_*p*_^0^ ) of the model (2), with respect to (*S*, *P*_*V*,_ *P*_*I*_, *T*, *R*) at the disease-free equilibrium point, we have the following characteristics equation.

(7) $$\begin{array}{c} \left(–\mu -\lambda_{1}\right)\left.\left(\left(r_{1}-r_{2}\right)-\lambda_{2}\right)\right)\;\left(-\left(\mu +\phi \right)-\lambda_{3}\right)\left(-\left(\beta +\mu \right)-\lambda_{4}\right)\left(-\left(Y+\mu \right)-\lambda_{5}\right)=0 \end{array}$$

Where  *r*_1_ = *ℛ*_*ef*(*p*)_ *r*_2_  and *r*_2_ = ( *τ*_2_ + *δ*_2_ + *μ*),

(8) $$\begin{array}{c} \Rightarrow \lambda_{1}=–\mu ,\lambda_{3}=-\left(\mu +\phi \right),\lambda_{4}=-\left(\beta +\mu \right),\lambda_{5}=-\left(Y+\mu \right). \end{array}$$

Hence, all the parameters are nonnegative, and all the eigenvalues of the corresponding Jacobean matrix are negative. But *λ*_2_ = (*r*_1_ − *r*_2_) = *ℛ*_*ef*(*p*)_ *r*_2_ − *r*_2_ = *r*_2_(*ℛ*_*ef*(*p*)_ − 1),

(9) $$\begin{array}{c} \Rightarrow \lambda_{2}=r_{2}\left(R_{ef\left(p\right)}-1\right), \end{array}$$

⇒*λ*_2_ < 0 *iff* *ℛ*_*ef*(*p*)_ < 1.Therefore, the disease-free equilibrium point is locally asymptotically stable if and only if *ℛ*_*ef*(*p*)_ < 1, otherwise it is unstable, that is, if *ℛ*_*ef*(*p*)_ > 1.

The article "Appraisal and Simulation on Codynamics of Pneumonia and Meningitis with Vaccination Intervention: From a Mathematical Model Perspective" was published in 2022. Journal: Comput Math Methods Med.

#### 2.3.2. Global Stability of Disease-Free Equilibrium Point of the Model

To verify the global stability of the disease-free equilibrium point of the pneumonia monoinfection model, we have used an adopted method of Castillo-Chavez et al. used by others scholar such as [18, 19].

**Lemma 1 .**

If the pneumonia monoinfection model can be written as

(10) $$\begin{array}{c} \frac{\text{dY}}{\text{dt}}=\text{G}\left(\text{Y},\text{W}\right),\\ \frac{dZ}{dt}=H\left(Y,W\right),H\left(Y,0\right)=0, \end{array}$$

where *Y* ∈ ℝ^*m*^ be the components of noninfected individuals and *W* ∈ ℝ^*n*^ be the components of infected individuals including treated class and *E*_*p*_^0^ = (*Y*^∗^, 0) denotes the disease-free equilibrium point of dynamical system (2).

Assume

- For  (*dY*/*dt*) = *G*(*Y*, 0),  *Y*^∗^ is globally asymptotically stable (GAS)
- $H\left(Y,W\right)=BW-\overset{ˇ}{H}\left(Y,W\right)$, $\;\overset{ˇ}{H}\left(Y,W\right)\geq 0$ for (*Y*, *W*) ∈ *Ω*_1_ where *B* = *D*_*W*_*H*(*Y*^∗^, 0) is an M-matrix, i.e., the off diagonal elements of *B* are nonnegative and *Ω*_1_ is the region in which the system makes biological sense. Then the fixed point *E*_*p*_^0^ = (*Y*^∗^, 0) is globally asymptotically stable equilibrium point of the system (2) whenever *R*_*ef*(*p*)_ < 1.

**Lemma 2 .**

The disease-free equilibrium point *E*_*p*_^0^  of the pneumonia monoinfection model (2) is globally asymptotically stable if *ℛ*_*ef*(*p*)_ < 1 and the two sufficient conditions given in Lemma 4 are satisfied.

Proof: here we are applying Lemma 5 on the pneumonia monoinfection model (2) and we have gotten the following matrices.

(11) $$\begin{array}{c} \frac{dY}{dt}=G\left(Y,W\right)=\left[\begin{array}{c} \left(1-\pi \right)\lambda +\phi \;P_{V}+YR–\left(\alpha_{2}+\mu \right)S\\ \pi \lambda -\left(\mu +\phi \right)P_{V} \end{array}\right],\\ \frac{dW}{dt}=H\left(Y,W\right)=\left[\begin{array}{c} \alpha_{2}S-\left(\tau_{2}+\delta_{2}+\mu \right)P_{I}\\ \tau_{2}P_{I}-\left(\beta +\mu \right)\text{T }\\ \beta T-\left(Y+\mu \right)R \end{array}\right],\\ G\left(Y,0\right)=\left[\begin{array}{c} \left(1-\pi \right)\lambda +\phi \;P_{V}-\mu S\\ \pi \lambda -\left(\mu +\phi \right)P_{V} \end{array}\right], \end{array}$$

and

(12) $$\begin{array}{c} \overset{ˇ}{H}\left(Y,W\right)=\left[\begin{array}{c} {\overset{ˇ}{H}}_{1}\left(Y,W\right)\\ {\overset{ˇ}{H}}_{2}\left(Y,W\right)\\ {\overset{ˇ}{H}}_{3}\left(Y,W\right) \end{array}\right]=\left[\begin{array}{c} \left(\frac{b\lambda }{\mu }\left(\frac{\left(1-\pi \right)\left(\mu +\phi \right)+\pi \phi }{\left(\mu +\phi \right)}\right)\right)P_{I}-\alpha_{2}S\\ 0\;\\ 0 \end{array}\right],\\ \overset{ˇ}{H}\left(Y,W\right)=\left[\begin{array}{c} {\overset{ˇ}{H}}_{1}\left(Y,W\right)\\ {\overset{ˇ}{H}}_{2}\left(Y,W\right)\\ {\overset{ˇ}{H}}_{3}\left(Y,W\right) \end{array}\right]=\left[\begin{array}{c} \left(S_{0}-S\right){bP}_{I}\\ 0\\ 0 \end{array}\right]. \end{array}$$

Since *S* ≤ *S*_0_, we have ${\overset{ˇ}{\;H}}_{1}\left(Y,W\right)\geq 0$, thus, the disease-free equilibrium point *E*_*p*_^0^ is globally asymptotically stable if  *ℛ*_*ef*(*p*)_ < 1. Biologically, whenever *ℛ*_*ef*(*p*)_ < 1, the only pneumonia infection disease dies out while the total population increases [18].

The article "Appraisal and Simulation on Codynamics of Pneumonia and Meningitis with Vaccination Intervention: From a Mathematical Model Perspective" was published in 2022. Journal: Comput Math Methods Med.

### 2.4. The Existence and Stability of Endemic Equilibrium Point

The endemic equilibrium point of the dynamical system of (2) is obtained by making the right side of the system equal to zero, providing that  *P*_*I*_ ≠ 0. We have supposed that the endemic equilibrium point of the model is denoted by  *E*_*p*_^∗^ = (*S*^∗^, *P*_*I*_^∗^, *P*_*v*_^∗^, T^∗^, R^∗^ ) and the corresponding force of infection is *α*_2_(t) = *b*(*P*_*I*_^∗^(t)).

For simplification of algebraic manipulation, we have assumed the parameters in the model by another variable as follows, *k*_1_ = (1 − *π*)*λ*, *k*_2_ = *τ*_2_ + *μ*, *k*_3_ = *τ*_2_ + *δ*_2_ + *μ*, *k*_4_ = *πλ*, *k*_5_ = *ϕ* + *μ*, 

*k*_6_ = *β* + *μ*, *k*_7_ = *Y* + *μ*, *k*_8_ = *γβτ*_2_, *k*_9_ = *k*_3_*k*_6_*k*_7_ ,  *k*_10_ = *k*_1_ + (*ϕk*_4_/*k*_5_),  *k*_11_ = *k*_9_*k*_10_, *k*_12_ = *k*_2_*k*_9_

*k*_13_ = *k*_3_*k*_12_ and *k*_14_ = *k*_8_*k*_3_. Now the equation of force of infection can be rearranged as

(13) $$\begin{array}{c} \;{\alpha_{2}}^{*}\left(k_{14}\;{\alpha_{2}}^{*}+bk_{11}-k_{13}\right)=0\Rightarrow {\alpha_{2}}^{*}=0\text{ or }k_{14}\;{\alpha_{2}}^{*}+bk_{11}-k_{13}=0, \end{array}$$

⇒*α*_2_^∗^ = *k*_13_ − *bk*_11_/*k*_14_ but  *α*_2_^∗^ = *k*_13_ − *bk*_11_/*k*_14_ = (*β* + *μ*)(*Y* + *μ*)((*τ*_2_ + *δ*_2_ + *μ*)(*τ*_2_ + *μ*)(*ϕ* + *μ*) − b*λ*((*ϕ* + *μ*)(1 − *π*) − *ϕπ*)/*γβτ*_2_(*ϕ* + *μ*)) = (*β* + *μ*)(*Y* + *μ*)((*τ*_2_ + *δ*_2_ + *μ*)(*τ*_2_ + *μ*)(*ϕ* + *μ*)/*γβτ*_2_(*ϕ* + *μ*) − *λ*b((*ϕ* + *μ*)(1 − *π*) + *ϕπ*)/*γβτ*_2_(*ϕ* + *μ*)), *α*_2_^∗^ = (*β* + *μ*)(*Y* + *μ*)((*τ*_2_ + *δ*_2_ + *μ*)(*τ*_2_ + *μ*)(*ϕ* + *μ*)/*γβτ*_2_)((*λb*/*μ*)((1 − *π*)(*μ* + *ϕ*) + *πϕ*/(*μ* + *ϕ*)(*τ*_2_ + *δ*_2_ + *μ*)) − 1)⇒*α*_2_^∗^ = (*β* + *μ*)(*Y* + *μ*)((*τ*_2_ + *δ*_2_ + *μ*)(*τ*_2_ + *μ*)(*ϕ* + *μ*)/*γβτ*_2_)( *ℛ*_*p*_ − 1)⇒*α*_2_^∗^ > 0 if *ℛ*_*ef*(*p*)_ > 1.

The article "Appraisal and Simulation on Codynamics of Pneumonia and Meningitis with Vaccination Intervention: From a Mathematical Model Perspective" was published in 2022. Journal: Comput Math Methods Med.

Therefore, there is a unique endemic equilibrium point for pneumonia monoinfected model as given by  *E*_*p*_^∗^ = (*S*^∗^, *P*_*I*_^∗^, *P*_*v*_^∗^, T^∗^, R^∗^ ) where

(14) $$\begin{array}{c} S^{*}=\frac{\left(\left(\tau_{2}+\delta_{2}+\mu \right)\left(\beta +\mu \right)\left(Y+\mu \right)\right)\left(\phi +\mu \right)-\left(\phi +\mu \right)\left(1-\pi \right)\lambda -\phi \pi \lambda }{\left(\phi +\mu \right)\left(\left(\tau_{2}+\mu \right)\left(\left(\tau_{2}+\delta_{2}+\mu \right)\left(\beta +\mu \right)\left(Y+\mu \right)\right)-\gamma \beta \tau_{2}{\alpha_{2}}^{*}\right)},\\ {P_{I}}^{*}=\frac{\left(\left(\tau_{2}+\delta_{2}+\mu \right)\left(\beta +\mu \right)\left(Y+\mu \right)\right)\left(\phi +\mu \right)-\left(\phi +\mu \right)\left(1-\pi \right)\lambda -\phi \pi \lambda }{\left(\phi +\mu \right)\left(\left(\tau_{2}+\mu \right)\left(\left(\tau_{2}+\delta_{2}+\mu \right)\left(\beta +\mu \right)\left(Y+\mu \right)\right)-\gamma \beta \tau_{2}{\alpha_{2}}^{*}\right)}\left(\frac{{\alpha_{2}}^{*}}{\tau_{2}+\delta_{2}+\mu }\right),{P_{v}}^{*}=\frac{\pi \lambda }{\phi +\mu },\\ {\text{T}}^{*}=\left(\frac{{\alpha_{2}}^{*}\tau_{2}}{\left(\tau_{2}+\delta_{2}+\mu \right)\left(\beta +\mu \right)}\right)\frac{\left(\left(\tau_{2}+\delta_{2}+\mu \right)\left(\beta +\mu \right)\left(Y+\mu \right)\right)\left(\phi +\mu \right)-\left(\phi +\mu \right)\left(1-\pi \right)\lambda -\phi \pi \lambda }{\left(\phi +\mu \right)\left(\left(\tau_{2}+\mu \right)\left(\left(\tau_{2}+\delta_{2}+\mu \right)\left(\beta +\mu \right)\left(Y+\mu \right)\right)-\gamma \beta \tau_{2}{\alpha_{2}}^{*}\right)},\\ R^{*}=\frac{\left(\left(\tau_{2}+\delta_{2}+\mu \right)\left(\beta +\mu \right)\left(Y+\mu \right)\right)\left(\phi +\mu \right)-\left(\phi +\mu \right)\left(1-\pi \right)\lambda -\phi \pi \lambda }{\left(\phi +\mu \right)\left(\left(\tau_{2}+\mu \right)\left(\left(\tau_{2}+\delta_{2}+\mu \right)\left(\beta +\mu \right)\left(Y+\mu \right)\right)-\gamma \beta \tau_{2}{\alpha_{2}}^{*}\right)}\left(\frac{\beta \tau_{2}{\alpha_{2}}^{*}}{\left(\tau_{2}+\delta_{2}+\mu \right)\left(\beta +\mu \right)\left(Y+\mu \right)}\right). \end{array}$$

**Theorem 4 .**

The article "Appraisal and Simulation on Codynamics of Pneumonia and Meningitis with Vaccination Intervention: From a Mathematical Model Perspective" was published in 2022. Journal: Comput Math Methods Med.

The endemic equilibrium point of system (2) *E*_*p*_^∗^ = (*S*^∗^, *P*_*I*_^∗^, *P*_*v*_^∗^, T^∗^, R^∗^ ) is locally asymptotically stable for the reproduction number *R*_*eff*(*p*)_ > 1.

Proof: to show that the local stability of the endemic equilibrium point, we have used the method of the Jacobian matrix and the Routh Hurwitz stability criteria.

Then the corresponding characteristic equation is obtained from the determinant of

(15) $$\begin{array}{c} \left|\begin{array}{ccccc} A-\lambda & \text{B} & C & 0 & D\\ E & F-\lambda & 0 & 0 & 0\\ 0 & 0 & \text{G}-\lambda & 0 & 0\\ 0 & \text{H} & 0 & I-\lambda & 0\\ 0 & 0 & 0 & J & K-\lambda \end{array}\right|=0, \end{array}$$

where *A* = –(*α*_2_*I*_*p*_^∗^ + *μ*), *B* = −*α*_2_*S*^∗^, *C* = *ϕ*, *D* = *Y*, *E* = *α*_2_*I*_*p*_^∗^, *F* = *α*_2_*S*^∗^ − ( *τ*_2_ + *δ*_2_ + *μ*),

(16) $$\begin{array}{c} G=-\left(\mu +\phi \right),H=\tau_{2},I=-\left(\beta +\mu \right),J=\beta \text{ and }k=-\left(Y+\mu \right),\\ \Rightarrow a_{0}\lambda^{5}+a_{1}\lambda^{4}+a_{2}\lambda^{3}+a_{3}\lambda^{2}+a_{4}\lambda +a_{5}=0, \end{array}$$

where  *a*_0_ = 1, −(*I* + *A* + *F* + *G* + *K*) = *a*_1_, (*IA* + IF + *AF* + *IG* + *AG* + *FG* + *IK* + *AK* + *FK* + *GK*) = *a*_2_, −(−*B* + *IAF* + *IAG* + *IFG* + *AFG* + *IAK* + *IFK* + *AFK* + *IGK* + *AGK* + *FGK*) = *a*_3_, −(*IB* − *IAFG* + *DEHJ* + *BK* − *IAFK* − *IAGK* − *IFGK* − *AFGK*) = *a*_4_, *a*_5_ = *DEGHJ* + *IBK* − *IAFGK*.

To apply the Routh-Hurwitz stability criteria, it is obligatory to check if the necessary condition of all the coefficients have the same sign or not. Since *a*_0_ = 1 is positive in sign, all  *a*_1_,  *a*_2_, *a*_3_, *a*_4_, and *a*_5_ should be positives in sign. All the coefficients of the characteristic's polynomial are positives whenever  *ℛ*_*eff*(*p*)_ > 1. We have observed that the first column of the Routh Hurwitz array has no sign change, thus the root of the characteristics equation of the dynamical system are negative. Hence, the endemic equilibrium point of the dynamical system is locally asymptotically stable.

### 2.5. Positivity of Solutions and Invariant Region of the Only Meningitis-Infected Model

We have made *P*_*I*_ = *MP*_*I*_ = 0 from the full pneumonia and meningitis coinfection model to obtain this submeningitis-only model, and got the following dynamical system.

(17) $$\begin{array}{c} \left.\begin{array}{c} \frac{dS}{dt}=\left(1-\pi \right)\lambda +\varphi M_{V}+YR–\left(\alpha_{1}+\mu \right)S,\\ \frac{dM_{I}}{dt}=\alpha_{1}S–\left(\;\tau_{1}+\delta_{1}+\mu \right)M_{I},\\ \;\frac{dM_{V}}{dt}=\pi \lambda -\left(\mu +\varphi \right)M_{V},\\ \frac{d\text{T}}{dt}=\tau_{1}M_{I}-\left(\beta +\mu \right)\text{T},\\ \frac{d\text{R}}{dt}=\beta T-\left(Y+\mu \right)R. \end{array}\right\} \end{array}$$

The above dynamical systems are needed to be epidemiologically meaningful as well as well-posed. To prove that, we have intimated that all the state variables of dynamical systems are nonnegative.

The article "Appraisal and Simulation on Codynamics of Pneumonia and Meningitis with Vaccination Intervention: From a Mathematical Model Perspective" was published in 2022. Journal: Comput Math Methods Med.

**Theorem 5 .**

All the populations of the system with positive initial conditions are positive.

Proof: assume *S*(0) > 0, *M*_*I*_(0) > 0, *M*_*V*_(0) > 0, *T*(0) > 0  and  *R*(0) > 0 are positive for time *t* > 0 and for all nonnegative. First let us take *T* = sup{*t* > 0 such that *S*(*t*′) > 0, *M*_*I*_(*t*′) > 0, *M*_*V*_(*t*′) > 0, *T*(*t*′) > 0 and *R*(*t*′) > 0, *t*′ ∈ [0, *t*]}.

From the first equation of system (17), we do have

(18) $$\begin{array}{c} \frac{dS}{dt}=\left(1-\pi \right)\lambda +\varphi M_{V}+YR–\left(\alpha_{1}+\mu \right)S,\\ S\left(t\right)=S\left(0\right)e^{-\int_{0}^{T}\left(\alpha_{1}+\mu \right)dt^{\prime }}+e^{-\int_{0}^{T}\left(\alpha_{1}+\mu \right)dt^{\prime }}\left[\int_{0}^{T}e^{\int_{0}^{T}\left(\alpha_{1}+\mu \right)dt^{\prime }}\left[\left(1-\pi \right)\lambda +YR+\varphi M_{V}\right.dt\right]>0,\\ \Rightarrow \text{S}\left(\text{t}\right)>0. \end{array}$$

Therefore, *S*(*t*) is positive. Subsequent to the same procedure, the remaining state variables are nonnegative. Therefore, from the stated proof, we can conclude that whenever the initial values of the systems are all nonnegative, then all the solutions of our dynamical system are positive.

**Theorem 6 .**

All the populations of the system with positive initial conditions are nonnegative

The total human population of the dynamical system (17) is positively closed in the closed invariant set *Ω*_2_ = {(*S*, *M*_*I*,_ *M*_*V*,_*T*, *R*)*ϵ*ℝ_+_^5^ : *N*_2_ ≤ *λ*/*μ*}. Furthermore, the system's nonnegative solutions are all constrained, and it may exhibit the persistence property under any nonnegative initial concentration conditions [14].

Proof: to get an invariant region, boundedness of solution is obtained as follow.

(19) $$\begin{array}{c} N_{2}=S+M_{I}+M_{V}+T+R,\\ \frac{dN_{2}}{dt}=\lambda -\mu N_{2}-\delta_{1}M_{I}\Rightarrow 0\leq N_{2}\leq \frac{\lambda }{\mu }. \end{array}$$

Therefore, the dynamical system that we do have is bounded.

### 2.6. Existence and Stability of Disease-Free Equilibrium Point

The disease-free equilibrium point is obtained by making all the equations in the system equal to zero, provided that providing that  *M*_*I*_ = 0. Therefore, the disease-free equilibrium point is

(20) $$\begin{array}{c} E_{p}^{0}=\left(S^{O},{M_{V}}^{O},{M_{I}}^{O},T^{0},R^{O}\;\right)=\left(\frac{\lambda }{\mu }\left[\frac{\left(1-\pi \right)\left(\mu +\varphi \right)+\pi \varphi }{\left(\mu +\varphi \right)}\right],\frac{\pi \lambda }{\left(\mu +\varphi \right)},0,0,0\right). \end{array}$$

The article "Appraisal and Simulation on Codynamics of Pneumonia and Meningitis with Vaccination Intervention: From a Mathematical Model Perspective" was published in 2022. Journal: Comput Math Methods Med.

#### 2.6.1. Effective Reproduction Number

The reproduction number can be defined as a number of secondary cases produced by one infectious individual joining in a completely susceptible population during its infectious period [16, 17, 20].

To compute the reproduction number, first distinguishing the new infected from all other changes in the host population is mandatory as follows.

Let  *ℱ*_*i*_(*x*): be the rate of appearance of new infected in compartment *i*,

*𝒱* ^+^_*i*_(*x*): be the rate of transfer of individuals in to compartment *i*, 

*𝒱* ^−^_*i*_(*x*): be the rate of transfer of individuals out of compartment *i*.

And then *𝒱*_*i*_(*x*) = *𝒱*^−^_*i*_(*x*) − *𝒱*^+^_*i*_ but *F* = [(*∂ℱ*_*i*_/*∂X*_*j*_)(*X*_*o*_)] and *V* = [(*∂𝒱*_*i*_/*∂X*_*j*_)(*X*_*o*_)], where *F* and V are *mxm* matrix with *m* is number of infected compartment. *Fv*^−1^ is the next generation matrix, and the spectral radius of next generation matrix is needed for the reproduction number we are seeking for.

Thus *∂ℱ*_*i*_(*X*)/*∂X*_*j*_ = *aS*  and  *∂𝒱*_*i*_(*X*)/*∂X*_*j*_ and  *FV*^−1^ = (*λa*/*μ*)((1 − *π*)(*μ* + *φ*) + *πφ*/(*μ* + *φ*)(*τ*_1_ + *δ*_1_ + *μ*))

Therefore, the effective reproduction number of meningitis monoinfected submodel is

(21) $$\begin{array}{c} R_{ef\left(m\right)}=\frac{\lambda a}{\mu }\left(\frac{\left(1-\pi \right)\left(\mu +\varphi \right)+\pi \varphi }{\left(\mu +\varphi \right)\left(\tau_{1}+\delta_{1}+\mu \right)}\right). \end{array}$$

**Theorem 7 .**

The disease-free equilibrium point  *E*_*m*_^0^ of the model in system (17) is locally asymptotically stable if the effective reproduction number *ℛ*_*ef*(*m*)_ < 1, and it is unstable if *ℛ*_*ef*(*m*)_ > 1.

Proof:

Using the Jacobean matrix  *J*(*E*_*p*_^0^ ) of the model (17) with respect to (*S*, *M*_*V*,_ *M*_*I*_, *T*, *R*) at the disease-free equilibrium point, we have the characteristic equation

(22) $$\begin{array}{c} \Rightarrow \left(–\mu -\lambda_{1}\right)\left.\left(\left(t_{1}-t_{2}\right)-\lambda_{2}\right)\right)\left(-\left(\mu +\varphi \right)\left.-\lambda_{3}\right)\left(-\left(\beta +\mu \right)-\lambda_{4}\right)\left(-\left(Y+\mu \right)-\lambda_{5}\right.\right)=0\text{ where }t_{1}=R_{ef\left(m\right)}\;t_{2}\text{ and }t_{2}=\left(\;\tau_{1}+\delta_{1}+\mu \right),\\ \Rightarrow \lambda_{1}=–\mu ,\lambda_{3}=-\left(\mu +\varphi \right),\lambda_{4}=-\left(\beta +\mu \right),\lambda_{5}=-\left(Y+\mu \right). \end{array}$$

Hence, all the parameters are nonnegative, all the eigenvalues of the corresponding Jacobean matrix are negative other than  *λ*_2_.

The article "Appraisal and Simulation on Codynamics of Pneumonia and Meningitis with Vaccination Intervention: From a Mathematical Model Perspective" was published in 2022. Journal: Comput Math Methods Med.

For *λ*_2_, *λ*_2_ = *t*_2_(*ℛ*_*eff*(*m*)_ − 1)⇒*λ*_2_ = *t*_2_(*ℛ*_*eff*(*m*)_ − 1),

(23) $$\begin{array}{c} \Rightarrow \lambda_{2}<0\text{ iff }R_{ef\left(m\right)}<1. \end{array}$$

Therefore, the disease-free equilibrium point of the meningitis monoinfected model is locally asymptotically stable if the effective reproduction number *ℛ*_*ef*(*m*)_ < 1 and is unstable if  *ℛ*_*ef*(*m*)_ > 1.

#### 2.6.2. Global Stability of Disease-Free Equilibrium Point

We utilized the approach developed by Castillo-Chavez et al. and used it to confirm the overall stability of the disease-free equilibrium point of the meningitis monoinfection model [18, 19].

**Lemma 3 .**

If the pneumonia monoinfection model can be written as

(24) $$\begin{array}{c} \frac{\text{dY}}{\text{dt}}=\text{G}\left(\text{Y},\text{W}\right),\\ \frac{dZ}{dt}=H\left(Y,W\right),H\left(Y,0\right)=0, \end{array}$$

where *Y* ∈ ℝ^*m*^ be the components of noninfected individuals and *W* ∈ ℝ^*n*^ be the components of infected individuals including the treated class, and  *E*_*m*_^0^ = (*Y*^∗^, 0) denotes the disease-free equilibrium point of the dynamical system (3).

Assume

- For  (*dY*/*dt*) = *G*(*Y*, 0), *Y*^∗^ is globally asymptotically stable (GAS)
- $H\left(Y,W\right)=BW-\overset{ˇ}{H}\left(Y,W\right)$, $\;\overset{ˇ}{H}\left(Y,W\right)\geq 0$ for (*Y*, *W*) ∈ *Ω*_1_ where *B* = *D*_*W*_*H*(*Y*^∗^, 0) is an M-matrix, i.e., the off diagonal elements of *B* are nonnegative and *Ω*_2_ is the region in which the system makes biological sense

Then the fixed point *E*_*m*_^0^ = (*Y*^∗^, 0) is globally asymptotically stable equilibrium point of the system (17) whenever *ℛ*_*ef*(*m*)_ < 1.

**Lemma 4 .**

The disease-free equilibrium point  *E*_*m*_^0^ of the pneumonia monoinfection model (17) is globally asymptotically stable if  *ℛ*_*ef*(*m*)_ < 1 and the two sufficient conditions given in Lemma 10 are satisfied.

Proof: here we are applying Lemma 11 on the meningitis monoinfection model (17) and we have gotten the following matrices $dY/dt=G\left(Y,W\right)=\left[\begin{array}{c} \left(1-\pi \right)\lambda +\varphi M_{V}+YR–\left(\alpha_{1}+\mu \right)S\\ \pi \lambda -\left(\mu +\varphi \right)M_{V}\; \end{array}\right],$

(25) $$\begin{array}{c} \frac{dW}{dt}=H\left(Y,W\right)=\left[\begin{array}{ccc} \frac{a\lambda }{\mu }\left(\frac{\left(1-\pi \right)\left(\mu +\phi \right)+\pi \phi }{\left(\mu +\phi \right)}\right)-\left(\;\tau_{1}+\delta_{1}+\mu \right) & 0 & 0\\ \tau_{1} & -\left(\beta +\mu \right) & 0\\ 0 & \beta & -\left(Y+\mu \right) \end{array}\right],\\ G\left(Y,0\right)=\left[\begin{array}{c} \left(1-\pi \right)\lambda +\varphi M_{V}-\mu S\\ \pi \lambda -\left(\mu +\varphi \right)M_{V}\; \end{array}\right]. \end{array}$$

Here after some steps of calculations, we have determined that

(26) $$\begin{array}{c} \overset{ˇ}{H}\left(Y,W\right)=\left[\begin{array}{c} {\overset{ˇ}{H}}_{1}\left(Y,W\right)\\ {\overset{ˇ}{H}}_{2}\left(Y,W\right)\\ {\overset{ˇ}{H}}_{3}\left(Y,W\right) \end{array}\right]=\left[\begin{array}{c} \left(S_{0}-S\right)aM_{I}\\ 0\;\\ 0 \end{array}\right]. \end{array}$$

Since *S* ≤ *S*_0_, we have ${\overset{ˇ}{\;H}}_{1}\left(Y,W\right)\geq 0$, thus, the disease-free equilibrium point  *E*_*m*_^0^ of model (17) is globally asymptotically stable if  *ℛ*_*ef*(*m*)_ < 1. Biologically, whenever  *ℛ*_*ef*(*m*)_ < 1, the meningitis monoinfection disease dies out while the total population increases [18].

The article "Appraisal and Simulation on Codynamics of Pneumonia and Meningitis with Vaccination Intervention: From a Mathematical Model Perspective" was published in 2022. Journal: Comput Math Methods Med.

### 2.7. Existence and Stability of Endemic Equilibrium Point

The endemic equilibrium point of the dynamical system of (3) is obtained by making the right side of the system equal to zero, providing that  *M*_*I*_ ≠ 0. We have supposed that the endemic equilibrium point of the model is denoted by  *E*_*m*_^∗^ = (*S*^∗^, *M*_*I*_^∗^, *M*_*v*_^∗^, T^∗^, R^∗^) and the corresponding force of infection is  *α*_1_(t) = *b*(*M*_*I*_^∗^(t)). For simplification of algebraic manipulation, we have assumed the parameters in the model by another variable as follows.

(27) $$\begin{array}{c} n_{1}=\left(1-\pi \right)\lambda ,n_{2}=\tau_{1}+\mu ,n_{3}=\left(\;\tau_{1}+\delta_{1}+\mu \right),n_{4}=\pi \lambda ,n_{5}=\left(\mu +\varphi \right),\\ n_{6}=\beta +\mu ,n_{7}=Y+\mu ,n_{8}=\gamma \beta \tau_{1},n_{9}=n_{3}n_{6}n_{7},n_{10}=n_{1}+\varphi n_{4}/n_{5},\;n_{11}=n_{9}n_{10},n_{12}=n_{2}n_{9}\; \end{array}$$

*n*_13_ = *n*_3_*n*_12_ and *n*_14_ = *n*_8_*n*_3_ . Now the equation of force of infection can be rearranged as

(28) $$\begin{array}{c} {\alpha_{1}}^{*}\left(n_{14}\;{\alpha_{1}}^{*}+an_{11}-n_{13}\right)=0\Rightarrow {\alpha_{1}}^{*}=0\text{ or }n_{14}\;{\alpha_{1}}^{*}+an_{11}-n_{13}=0\\ \Rightarrow {\alpha_{1}}^{*}=\frac{n_{13}-{\text{an}}_{11}}{n_{14}},\text{but }{\alpha_{1}}^{*}=\frac{n_{13}-{\text{an}}_{11}}{n_{14}}=\left(\beta +\mu \right)\left(Y+\mu \right)\left(\frac{\left(\tau_{1}+\delta_{1}+\mu \right)\left(\tau_{1}+\mu \right)\left(\varphi +\mu \right)-\text{a}\lambda \left(\left(\varphi +\mu \right)\left(1-\pi \right)-\varphi \pi \right)}{\gamma \beta \tau_{1}\left(\varphi +\mu \right)}\right)=\left(\beta +\mu \right)\left(Y+\mu \right)\left(\frac{\left(\tau_{1}+\delta_{1}+\mu \right)\left(\tau_{1}+\mu \right)\left(\varphi +\mu \right)}{\gamma \beta \tau_{2}\left(\phi +\mu \right)}-\frac{\lambda \text{a}\left(\left(\varphi +\mu \right)\left(1-\pi \right)+\varphi \pi \right)}{\gamma \beta \tau_{1}\left(\varphi +\mu \right)}\right),\\ {\alpha_{1}}^{*}=\left(\beta +\mu \right)\left(Y+\mu \right)\left(\frac{\left(\tau_{1}+\delta_{1}+\mu \right)\left(\tau_{1}+\mu \right)\left(\varphi +\mu \right)}{\gamma \beta \tau_{1}}\right)\left(\frac{\lambda a}{\mu }\left(\frac{\left(1-\pi \right)\left(\varphi +\mu \right)+\pi \varphi }{\left(\varphi +\mu \right)\left(\tau_{1}+\delta_{1}+\mu \right)}\right)-1\right),\\ \Rightarrow {\alpha_{1}}^{*}=\left(\beta +\mu \right)\left(Y+\mu \right)\left(\frac{\left(\tau_{1}+\delta_{1}+\mu \right)\left(\tau_{1}+\mu \right)\left(\varphi +\mu \right)}{\gamma \beta \tau_{1}}\right)\left(R_{eff\left(m\right)}-1\right)\Rightarrow {\alpha_{1}}^{*}>0\text{ if }R_{eff\left(m\right)}>1. \end{array}$$

Therefore, the unique endemic equilibrium point for the meningitis monoinfected model is given by  *E*_*m*_^∗^ = (*S*^∗^, *M*_*I*_^∗^, *M*_*v*_^∗^, T^∗^, R^∗^ ), where

(29) $$\begin{array}{c} S^{*}=\frac{\left(\left(\tau_{1}+\delta_{1}+\mu \right)\left(\beta +\mu \right)\left(Y+\mu \right)\right)\left(\varphi +\mu \right)-\left(\varphi +\mu \right)\left(1-\pi \right)\lambda -\varphi \pi \lambda }{\left(\varphi +\mu \right)\left(\left(\tau_{1}+\mu \right)\left(\left(\tau_{1}+\delta_{1}+\mu \right)\left(\beta +\mu \right)\left(Y+\mu \right)\right)-\gamma \beta \tau_{1}{\alpha_{1}}^{*}\right)},\\ {M_{I}}^{*}=\frac{\left(\left(\tau_{1}+\delta_{1}+\mu \right)\left(\beta +\mu \right)\left(Y+\mu \right)\right)\left(\varphi +\mu \right)-\left(\varphi +\mu \right)\left(1-\pi \right)\lambda -\varphi \pi \lambda }{\left(\varphi +\mu \right)\left(\left(\tau_{1}+\mu \right)\left(\left(\tau_{1}+\delta_{1}+\mu \right)\left(\beta +\mu \right)\left(Y+\mu \right)\right)-\gamma \beta \tau_{1}{\alpha_{1}}^{*}\right)}\left(\frac{{\alpha_{1}}^{*}}{\left(\tau_{1}+\delta_{1}+\mu \right)}\right),\\ {M_{v}}^{*}=\frac{\pi \lambda }{\left(\varphi +\mu \right)},\\ {\text{T}}^{*}=\left(\frac{{\alpha_{1}}^{*}\tau_{1}}{\left(\tau_{1}+\delta_{1}+\mu \right)\left(\beta +\mu \right)}\right)\frac{\left(\left(\tau_{1}+\delta_{1}+\mu \right)\left(\beta +\mu \right)\left(Y+\mu \right)\right)\left(\varphi +\mu \right)-\left(\varphi +\mu \right)\left(1-\pi \right)\lambda -\varphi \pi \lambda }{\left(\varphi +\mu \right)\left(\left(\tau_{1}+\mu \right)\left(\left(\tau_{1}+\delta_{1}+\mu \right)\left(\beta +\mu \right)\left(Y+\mu \right)\right)-\gamma \beta \tau_{1}{\alpha_{1}}^{*}\right)},\\ R^{*}=\frac{\left(\left(\tau_{1}+\delta_{1}+\mu \right)\left(\beta +\mu \right)\left(Y+\mu \right)\right)\left(\varphi +\mu \right)-\left(\varphi +\mu \right)\left(1-\pi \right)\lambda -\varphi \pi \lambda }{\left(\varphi +\mu \right)\left(\left(\tau_{2}+\mu \right)\left(\left(\tau_{1}+\delta_{1}+\mu \right)\left(\beta +\mu \right)\left(Y+\mu \right)\right)-\gamma \beta \tau_{2}{\alpha_{2}}^{*}\right)}\left(\frac{\beta \tau_{2}{\alpha_{2}}^{*}}{\left(\tau_{1}+\delta_{1}+\mu \right)\left(\beta +\mu \right)\left(Y+\mu \right)}\right). \end{array}$$

**Theorem 8 .**

The article "Appraisal and Simulation on Codynamics of Pneumonia and Meningitis with Vaccination Intervention: From a Mathematical Model Perspective" was published in 2022. Journal: Comput Math Methods Med.

The endemic equilibrium point of system (17) *E*_*m*_^∗^ = (*S*^∗^, *M*_*I*_^∗^, *M*_*v*_^∗^, T^∗^, R^∗^ ) is locally asymptotically stable for the reproduction number *R*_*eff*(*m*)_ > 1.

Proof: To show the local stability of the endemic equilibrium point we have used the method of Jacobian matrix and Routh Hurwitz stability criteria.

From Jacobian matrix, we have obtained the following characteristic equation

(30) $$\begin{array}{c} \left(a-\lambda \right)\left(f-\lambda \right)\left(\text{g}-\lambda \right)\left(i-\lambda \right)\left(k-\lambda \right)-\text{b}\left(i-\lambda \right)\left(k-\lambda \right)-d\text{e}\left(\text{g}-\lambda \right)hj=0 \end{array}$$

Where *a* = –(*α*_1_*I*_*m*_^∗^ + *μ*), *b* = −*α*_1_*S*^∗^, *c* = *φ*, *d* = *Y*, *e* = *α*_1_*I*_*m*_^∗^, *f* = *α*_1_*S*^∗^ − ( *τ*_1_ + *δ*_1_ + *μ*),

(31) $$\begin{array}{c} g=-\left(\mu +\varphi \right),h=\tau_{1},i=-\left(\beta +\mu \right),j=\beta \text{ and }k=-\left(Y+\mu \right).\\ \Rightarrow a_{0}\lambda^{5}+a_{1}\lambda^{4}+a_{2}\lambda^{3}+a_{3}\lambda^{2}+a_{4}\lambda +a_{5}=0 \end{array}$$

Where  *a*_0_ = 1, −(*i* + *a* + *f* + *g* + *k*) = *a*_1_, (*ai* + if + *af* + *ig* + *ag* + *fg* + *ik* + *ak* + *fk* + *g*) = *a*_2_, −(−*b* + *aif* + *aig* + *ifg* + *afg* + *aik* + *ifk* + *afk* + *gik* + *agk* + *fgk*) = *a*_3_, −(*bi* − *aifg* + *dehj* + *bk* − *aifk* − *aigk* − *ifgk* − *afgk*) = *a*_4_

*a*_5_ = *aeghj* + *bik* − *aifgk*.

To apply Routh-Hurwitz stability criteria, it is the must to check the necessary condition of all the coefficients have the same sign or not. Since *a*_0_ = 1 is positive in sign, all  *a*_1_,  *a*_2_, *a*_3_, *a*_4_ and *a*_5_ should be positives in sign. All the coefficients of the characteristic's polynomial are positives whenever *ℛ*_*eff*(*p*)_ > 1.

We have observed that the first column of the Routh Hurwitz array has no sign change, thus the root of the characteristics equation of the dynamical system  *a*_0_*λ*^5^ + *a*_1_*λ*^4^ + *a*_2_*λ*^3^ + *a*_3_*λ*^2^ + *a*_4_*λ* + *a*_5_ = 0 are negative. Hence, the endemic equilibrium point of the dynamical system is locally asymptotically stable.

The article "Appraisal and Simulation on Codynamics of Pneumonia and Meningitis with Vaccination Intervention: From a Mathematical Model Perspective" was published in 2022. Journal: Comput Math Methods Med.

### 2.8. Positivity and Boundedness of Full Pneumonia and Meningitis Coinfected Model

The corresponding dynamical system of the full pneumonia and meningitis coinfection model is given in Equation (1).

The constructed model is expected to be meaningful epidemiologically as well as well-posed. We need to prove that all the state variables of the dynamical system are positive.

**Theorem 9 .**

All the population of the system with positive initial conditions are nonnegative

Proof: Assume  *S*(0) > 0, *M*_*V*_(0) > 0, *P*_*V*_(0) > 0, *MP*_*V*_(0) > 0 , *M*_*I*_(0) > 0, *P*_*I*_(0) > 0, *MP*_*I*_(0) > 0 T(0) > 0, and  *R*(0) > 0 are positive for time *t* > 0 and for all nonnegative parameters. Let us define  *τ* = sup{*t* > 0 such that *S*(*t*) > 0, *M*_*V*_(*t*) > 0, *P*_*V*_(*t*) > 0, *MP*_*V*_(*t*) > 0, *M*_*I*_(*t*) > 0, *P*_*I*_(*t*) > 0, *MP*_*I*_(*t*) > 0, T(*t*) > 0, *R*(*t*) > 0 and *t* ∈ [0, *t*]}.

Since all  *S*(*t*), *M*_*V*_(*t*), *P*_*V*_(*t*), *MP*_*V*_(*t*), *M*_*I*_(*t*), *P*_*I*_(*t*), *MP*_*I*_(*t*), T(*t*) and *R*(*t*) are continuous, we can say for *τ* > 0. If *τ* = +∞, then positivity holds.

Nevertheless, if  0 < *τ* < +∞, then all the state variables are zeros.

From the first equation of system (1) we do have

(32) $$\begin{array}{c} \frac{dS}{dt}=\left(1-\pi \right)\lambda +\phi \;P_{V}+\varphi M_{V}+YR–\left(\alpha_{1}+\alpha_{2}+\mu \right)S\;S\left(t\right)=S\left(0\right)e^{-\int_{0}^{\tau }\left(\alpha_{1}+\alpha_{2}+\mu \right)dt}+e^{-\int_{0}^{\tau }\left(\alpha_{1}+\alpha_{2}+\mu \right)dt}\left[\int_{0}^{\tau }e^{\int_{0}^{\tau }\left(\alpha_{1}+\alpha_{2}+\mu \right)dt}\left(\left(1-\pi \right)\lambda +\phi \;P_{V}+\varphi M_{V}+YR\right)dt\right]>0\Rightarrow S\left(t\right)>0 \end{array}$$

Following same procedure, all the remaining state variables are nonnegative.

Therefore, from proof, we can conclude that whenever the initial values of the systems are all nonnegative, then all the solutions of our dynamical system are positive.

**Theorem 10 .**

The total human population is assumed to be *N* and the dynamical system (1) is positively invariant in the closed invariant set  *Ω* = {(*S*, *M*_*V*_, *P*_*V*,_ *MP*_*V*,_ *M*_*I*,_ *P*_*I*,_*MP*_*I*,_*T*, *R*)*ϵ*ℝ_+_^9^ : *N* ≤ *λ*/*μ*}. Furthermore, the system's nonnegative solutions are all constrained, and it may exhibit the persistence property under any nonnegative initial concentration conditions [24]. Proof: to get an invariant region, which shows boundedness of solution, is obtained as follow.

(33) $$\begin{array}{c} \frac{dN}{dt}=\frac{dS}{dt}+\frac{dM_{V}}{dt}+\frac{dP_{V}}{dt}+\frac{d{MP}_{V}}{dt}+\frac{dM_{I}}{dt}+\frac{dP_{I}}{dt}+\frac{d{MP}_{I}}{dt}+\frac{dT}{dt}+\frac{dR}{dt}, \end{array}$$

(34) $$\begin{array}{c} \Rightarrow \frac{\text{dN}}{\text{dt}}=\lambda -\mu \text{N}-\delta_{2}{\text{P}}_{\text{I}}-\delta_{1}{\text{M}}_{\text{I}}-\delta_{3}{\text{MP}}_{\text{I}}, \end{array}$$

(35) $$\begin{array}{c} \Rightarrow N\left(t\right)\leq N_{0}e^{-\mu t}+\frac{\lambda }{\mu }\Rightarrow 0\leq N\leq \frac{\lambda }{\mu }. \end{array}$$

Therefore, the dynamical system that we have constructed is bounded.

The article "Appraisal and Simulation on Codynamics of Pneumonia and Meningitis with Vaccination Intervention: From a Mathematical Model Perspective" was published in 2022. Journal: Comput Math Methods Med.

### 2.9. Disease-Free Equilibrium Point and Its Stability

The disease-free equilibrium point of full pneumonia and meningitis coinfection model *E*_*pm*_^*O*^ is obtained by making all the right-hand-side of equation in system (1), providing that all the infectious classes are equal to zero.

(36) $$\begin{array}{c} \left(S^{O},{M_{V,}}^{O}\;{P_{V}}^{O},{{MP}_{V}}^{0},{M_{I}}^{0},{P_{I}}^{0},{{MP}_{I}}^{0},T^{0},R^{O}\right)=\left(\frac{\left(1-\pi \right)\lambda }{\left(\alpha_{1}+\alpha_{2}+\mu \right)}+\left(\frac{\pi \lambda }{\left(\alpha_{1}+\alpha_{2}+\mu \right)}\right)\;\left(\frac{\phi \rho }{\left(\mu +\phi +\varepsilon_{2}\right)}+\frac{\left(1-\rho \right)\varphi }{\left(\mu +\varphi +\varepsilon_{1}\right)}\right),\frac{\left(1-\rho \right)\pi \lambda }{\left(\mu +\varphi +\varepsilon_{1}\right)},\frac{\rho \pi \lambda }{\left(\mu +\phi +\varepsilon_{2}\right)},\frac{\left(1-\rho \right)\pi \lambda \varepsilon_{1}}{\mu \left(\mu +\varphi +\varepsilon_{1}\right)}+\frac{\rho \pi \lambda \varepsilon_{2}}{\mu \left(\mu +\phi +\varepsilon_{2}\right)},0,0,0,0,0\;\right) \end{array}$$

#### 2.9.1. Effective Reproduction Number

The reproduction number is the average number of people that become infected because of the entry of one infectious person into a completely susceptible population in the absence of intervention. Moreover, reproduction number is utilized to determine the effect of the control measures and to understand the capability of the spread of the infection to disseminate in the entire community when the control strategies are applied [15, 17, 21].

The reproduction number of pneumonia and meningitis confection model denoted by *ℛ*_*eff*_, which is manipulated by the Van den Driesch, Pauline, and James Warmouth next generation matrix approach [20], is the largest eigenvalue of the next generation matrix *FV*^−1^ = [*∂ℱ*_*i*_( *E*_*r*_^*O*^)/*∂x*_*j*_][*∂ν*_*i*_( *E*_*r*_^*O*^)/*∂x*_*j*_]^−1^ , where  *ℱ*_*i*_  is the rate of appearance of new infection in compartment  *i* , *ν*_*i*_  is the transfer of infections from one compartment *i*  to another, and *E*_*pm*_^0^ is the disease-free equilibrium point.

The

(37) $$\begin{array}{c} F_{\text{i}}\left(\text{x}\right)=\left[\begin{array}{c} \alpha_{1}{\text{S}}^{\text{O}}\\ \alpha_{2}{\text{S}}^{\text{O}}\\ 0\\ 0\\ 0\\ 0\\ 0\\ 0\\ 0 \end{array}\right],\\ \nu_{i}=\left[\begin{array}{c} \left(\pi -1\right)\lambda -\phi \;{P_{V}}^{O}-\varphi {M_{V}}^{O}-YR^{0}+\mu S^{O}\;\\ \left(\mu +\varphi +\varepsilon_{1}\right){M_{V}}^{O}-\left(1-\rho \right)\pi \lambda \\ \left(\mu +\phi +\varepsilon_{2}\right){P_{V}}^{O}-\rho \pi \lambda \\ \mu {{MP}_{V}}^{0}-\varepsilon_{1}{M_{V}}^{O}-\varepsilon_{2}{P_{V}}^{O}\\ \left(\;\omega_{2}\alpha_{2}+\tau_{1}+\delta_{1}+\mu \right){M_{I}}^{0}\\ \left(\;\omega_{1}\alpha_{1}+\tau_{2}+\delta_{2}+\mu \right){P_{I}}^{0}\\ \left(\tau_{3}+\mu \right){{MP}_{I}}^{0}-\omega_{1}\alpha_{1}P_{I}-\omega_{2}\alpha_{2}{M_{I}}^{0}\\ \left(\beta +\mu \right)\text{T}-\tau_{1}{M_{I}}^{0}-\tau_{2}P_{I}-\tau_{3}{{MP}_{I}}^{0}\\ \left(Y+\mu \right)R^{0}-\beta T^{0} \end{array}\right]. \end{array}$$

Then

(38) $$\begin{array}{c} F=\left[\frac{\left(1-\pi \right)\lambda }{\mu }+\left(\frac{\pi \lambda }{\mu }\right)\;\left(\frac{\phi \rho }{\left(\mu +\phi +\varepsilon_{2}\right)}+\frac{\left(1-\rho \right)\varphi }{\left(\mu +\varphi +\varepsilon_{1}\right)}\right)\right]\left[\begin{array}{ccc} a & 0 & a\\ 0 & b & b\\ 0 & 0 & 0 \end{array}\right], \end{array}$$

and

(39) $$\begin{array}{c} V=\left[\begin{array}{ccc} \left(\;\tau_{1}+\delta_{1}+\mu \right) & 0 & 0\\ 0 & \left(\tau_{2}+\delta_{2}+\mu \right) & 0\\ 0 & 0 & \left(\tau_{3}+\mu \right) \end{array}\right]\Rightarrow FV^{-1}=\left[\begin{array}{ccc} \frac{a}{\left(\;\tau_{1}+\delta_{1}+\mu \right)} & 0 & \frac{a}{\left(\tau_{3}+\mu \right)}\\ 0 & \frac{b}{\left(\tau_{2}+\delta_{2}+\mu \right)} & \frac{b}{\left(\tau_{3}+\mu \right)}\\ 0 & 0 & 0 \end{array}\right]. \end{array}$$

The eigenvalues of the next generation matrix *F*.*V*^−1^ are

(40) $$\begin{array}{c} \left\{0,\frac{a\lambda \left(1-\pi \right)}{\left(\;\tau_{1}+\delta_{1}+\mu \right)\left(\mu \right)}+\frac{\phi \rho \left(\mu +\varphi +\varepsilon_{1}\right)+\varphi \left(1-\rho \right)\left(\mu +\phi +\varepsilon_{2}\right)}{\left(\mu +\phi +\varepsilon_{2}\right)\left(\mu \right)}\left(\frac{\pi \lambda a}{\tau_{1}+\delta_{1}+\mu }\right),\frac{b\lambda \left(1-\pi \right)}{\left(\;\tau_{2}+\delta_{2}+\mu \right)\left(\mu \right)}+\frac{\phi \rho \left(\mu +\varphi +\varepsilon_{1}\right)+\varphi \left(1-\rho \right)\left(\mu +\phi +\varepsilon_{2}\right)}{\left(\mu +\phi +\varepsilon_{2}\right)\left(\mu \right)}\left(\frac{\pi \lambda b}{\tau_{2}+\delta_{2}+\mu }\right)\right\}. \end{array}$$

Therefore, the effective reproduction number of full meningitis and pneumonia model is

(41) $$\begin{array}{c} \;R_{eff}=\max\left\{\frac{a\lambda \left(1-\pi \right)}{\left(\;\tau_{1}+\delta_{1}+\mu \right)\mu }+\frac{\phi \rho \left(\mu +\varphi +\varepsilon_{1}\right)+\varphi \left(1-\rho \right)\left(\mu +\phi +\varepsilon_{2}\right)}{\left(\mu +\phi +\varepsilon_{2}\right)\mu }\left(\frac{\pi \lambda a}{\tau_{1}+\delta_{1}+\mu }\right),\frac{b\lambda \left(1-\pi \right)}{\left(\;\tau_{2}+\delta_{2}+\mu \right)\mu }+\frac{\phi \rho \left(\mu +\varphi +\varepsilon_{1}\right)+\varphi \left(1-\rho \right)\left(\mu +\phi +\varepsilon_{2}\right)}{\left(\mu +\phi +\varepsilon_{2}\right)\mu }\left(\frac{\pi \lambda b}{\tau_{2}+\delta_{2}+\mu }\right)\right\}, \end{array}$$

*ℛ*_*eff*_ = max{*R*_1_, *R*_2_} where  *R*_1_ = *aλ*(1 − *π*)/( *τ*_1_ + *δ*_1_ + *μ*)*μ* + (*ϕρ*(*μ* + *φ* + *ε*_1_) + *φ*(1 − *ρ*)(*μ* + *ϕ* + *ε*_2_))/(*μ* + *ϕ* + *ε*_2_)*μ*(*πλa*/*τ*_1_ + *δ*_1_ + *μ*), and *R*_2_ = *bλ*(1 − *π*)/( *τ*_2_ + *δ*_2_ + *μ*)*μ* + (*ϕρ*(*μ* + *φ* + *ε*_1_) + *φ*(1 − *ρ*)(*μ* + *ϕ* + *ε*_2_)/(*μ* + *ϕ* + *ε*_2_)*μ*)(*πλb*/(*τ*_2_ + *δ*_2_ + *μ*)).

The article "Appraisal and Simulation on Codynamics of Pneumonia and Meningitis with Vaccination Intervention: From a Mathematical Model Perspective" was published in 2022. Journal: Comput Math Methods Med.

**Theorem 11 .**

The disease-free equilibrium point *E*_*pm*_^*O*^ of the model in system (17) is locally asymptotically stable if the effective reproduction number *ℛ*_*eff*_ < 1 and is unstable if *ℛ*_*eff*_ > 1.

Proof:

The Jacobean matrix *J*(*E*_*pm*_^*O*^ ) of the model (1) with respect to (*S*, *M*_*V*,_ *P*_*V*_, *MP*_*V*_, *M*_*I*_, *P*_*I*_, *MP*_*I*_, *T*, *R*) at the disease-free equilibrium point is the following:

(42) $$\begin{array}{c} J\left({E_{pm}}^{O}\right)=\left[\begin{array}{ccccccccc} –\mu & \varphi & \phi & 0 & r_{1} & r_{2} & r_{3} & 0 & Y\\ 0 & r_{4} & 0 & 0 & 0 & 0 & 0 & 0 & 0\\ 0 & 0 & r_{5} & 0 & 0 & 0 & 0 & 0 & 0\\ 0 & \varepsilon_{1} & \varepsilon_{2} & -\mu & 0 & 0 & 0 & 0 & 0\\ 0 & 0 & 0 & 0 & r_{6} & 0 & 0 & 0 & 0\\ 0 & 0 & 0 & 0 & 0 & r_{7} & 0 & 0 & 0\\ 0 & 0 & 0 & 0 & 0 & 0 & r_{8} & 0 & 0\\ 0 & 0 & 0 & 0 & \tau_{1} & \tau_{2} & \tau_{3} & r_{9} & 0\\ 0 & 0 & 0 & 0 & 0 & 0 & 0 & \beta & r_{10} \end{array}\right], \end{array}$$

where

(43) $$\begin{array}{c} r_{1}=-a\left(\left(\left(1-\pi \right)\lambda /\mu \right)+\left(\pi \lambda /\mu \right)\;\left(\left(\phi \rho /\left(\mu +\phi +\varepsilon_{2}\right)\right)+\left(\left(1-\rho \right)\varphi /\left(\mu +\varphi +\varepsilon_{1}\right)\right)\right)\right),r_{2}=-b\left(\left(1-\pi \right)\lambda /\left(\alpha_{1}+\alpha_{2}+\mu \right)+\left(\pi \lambda /\mu \right)\;\left(\left(\phi \rho /\left(\mu +\phi +\varepsilon_{2}\right)\right)+\left(\left(1-\rho \right)\varphi /\left(\mu +\varphi +\varepsilon_{1}\right)\right)\right)\right),r_{3}=-\left(a{ℯ}_{1}+b{ℯ}_{2}\right)\left(\left(\left(1-\pi \right)\lambda /\mu \right)+\left(\pi \lambda /\mu \right)\;\left(\left(\phi \rho /\left(\mu +\phi +\varepsilon_{2}\right)\right)+\left(\left(1-\rho \right)\varphi /\left(\mu +\varphi +\varepsilon_{1}\right)\right)\right)\right),r_{4}=-\left(\mu +\varphi +\varepsilon_{1}\right),r_{5}=-\left(\mu +\phi +\varepsilon_{2}\right),r_{6}=a\left(\frac{\left(1-\pi \right)\lambda }{\mu }+\left(\frac{\pi \lambda }{\mu }\right)\;\left(\frac{\phi \rho }{\left(\mu +\phi +\varepsilon_{2}\right)}+\frac{\left(1-\rho \right)\varphi }{\left(\mu +\varphi +\varepsilon_{1}\right)}\right)\right)–\left(\;\tau_{1}+\delta_{1}+\mu \right),r_{7}=b\left(\frac{\left(1-\pi \right)\lambda }{\mu }+\left(\frac{\pi \lambda }{\mu }\right)\;\left(\frac{\phi \rho }{\left(\mu +\phi +\varepsilon_{2}\right)}+\frac{\left(1-\rho \right)\varphi }{\left(\mu +\varphi +\varepsilon_{1}\right)}\right)\right)-\left(\tau_{2}+\delta_{2}+\mu \right),\\ \;r_{8}=-\left(\tau_{3}+\mu \right),r_{9}=-\left(\beta +\mu \right)\text{ and }r_{10}=-\left(Y+\mu \right)\Rightarrow \left(\lambda_{1}+\mu \right)\left(\lambda_{4}+\mu \right)\left(-\lambda_{2}+r_{4}\right)\left(-\lambda_{3}+r_{5}\right)\left(-\lambda_{5}+r_{6}\right)\left(-\lambda_{6}+r_{7}\right)\left(-\lambda_{7}+r_{8}\right)\left(-\lambda_{8}+r_{9}\right)\left(-\lambda_{9}+r_{10}\right)\Rightarrow \lambda_{1}=-\mu ,\lambda_{4}=-\mu ,\lambda_{2}=r_{4}=-\left(\mu +\varphi +\varepsilon_{1}\right),\lambda_{3}=r_{5}=-\left(\mu +\phi +\varepsilon_{2}\right),\lambda_{7}=r_{8}=-\left(\tau_{3}+\mu \right),\lambda_{8}=r_{9}=-\left(\beta +\mu \right)\;,\\ \lambda_{5}=\left(\;\tau_{1}+\delta_{1}+\mu \right)\;\left[\left(\frac{a\lambda \left(\mu +\varphi \right)}{\mu \left(1-\pi \right)\left(\mu +\varphi \right)+\pi \varphi }\right)\left(\;\frac{\left(\mu +\phi +\varepsilon_{2}\right)+\pi \phi \rho }{\left(\mu +\phi +\varepsilon_{2}\right)}+\frac{\left(1-\rho \right)\pi \varphi }{\left(\mu +\varphi +\varepsilon_{1}\right)}\right)\left(\left(\frac{a\lambda \left(1-\pi \right)\left(\mu +\varphi \right)+\pi \varphi }{\mu \left(\mu +\varphi \right)\left(\;\tau_{1}+\delta_{1}+\mu \right)\;}\right)-1\right)\right]\Rightarrow \lambda_{5}=\left(\;\tau_{1}+\delta_{1}+\mu \right)\;\left[\left(\frac{a\lambda \left(\mu +\varphi \right)}{\mu \left(1-\pi \right)\left(\mu +\varphi \right)+\pi \varphi }\right)\left(\;\frac{\left(\mu +\phi +\varepsilon_{2}\right)+\pi \phi \rho }{\left(\mu +\phi +\varepsilon_{2}\right)}+\frac{\left(1-\rho \right)\pi \varphi }{\left(\mu +\varphi +\varepsilon_{1}\right)}\right)\left(R_{eff\left(m\right)}-1\right)\right].\\ \lambda_{6}=\left(\tau_{2}+\delta_{2}+\mu \right)\left[\left(\frac{b\lambda \left(\mu +\phi \right)}{\mu \left(1-\pi \right)\left(\mu +\phi \right)+\pi \varphi }\right)\left(\;\frac{\left(\mu +\phi +\varepsilon_{2}\right)+\pi \phi \rho }{\left(\mu +\phi +\varepsilon_{2}\right)}+\frac{\left(1-\rho \right)\pi \varphi }{\left(\mu +\varphi +\varepsilon_{1}\right)}\right)\left(\frac{\lambda b}{\mu }\left(\frac{\left(1-\pi \right)\left(\mu +\phi \right)+\pi \phi }{\left(\mu +\phi \right)\left(\tau_{2}+\delta_{2}+\mu \right)}\right)\right)-1\right]\Rightarrow \lambda_{6}=\left(\tau_{2}+\delta_{2}+\mu \right)\left[\left(\frac{b\lambda \left(\mu +\phi \right)}{\mu \left(1-\pi \right)\left(\mu +\phi \right)+\pi \varphi }\right)\left(\;\frac{\left(\mu +\phi +\varepsilon_{2}\right)+\pi \phi \rho }{\left(\mu +\phi +\varepsilon_{2}\right)}+\frac{\left(1-\rho \right)\pi \varphi }{\left(\mu +\varphi +\varepsilon_{1}\right)}\right)\left(R_{eff\left(p\right)}-1\right)\right]\text{ and }\lambda_{9}=r_{10}=-\left(Y+\mu \right). \end{array}$$

Hence, all the parameters are nonnegative as well as all the eigenvalues of the corresponding Jacobean matrix are negative except *λ*_5_ and *λ*_6_.

The article "Appraisal and Simulation on Codynamics of Pneumonia and Meningitis with Vaccination Intervention: From a Mathematical Model Perspective" was published in 2022. Journal: Comput Math Methods Med.

The sign of eigenvalues *λ*_5_ and *λ*_6_ depends on the values of *R*_*eff*(*m*)_ and *R*_*eff*(*p*)_, respectively. Moreover,  *λ*_5_ < 0 whenever *R*_*eff*(*m*)_ < 1  and *λ*_6_ < 0 if and only if  *R*_*eff*(*p*)_ < 1.

Therefore, the disease-free equilibrium point of the full meningitis and pneumonia coinfection model is local asymptotically stable only if *R*_*eff*(*m*)_ < 1  and  *R*_*eff*(*p*)_ < 1 , otherwise it is unstable.

#### 2.9.2. Global Stability of Disease-Free Equilibrium Point

The disease-free equilibriums of the meningitis monoinfection model and the pneumonia monoinfection model are both globally asymptotically stable whenever their corresponding effective reproduction numbers values are smaller than unity, as demonstrated in Section 3Figure 2 and 3, respectively. In light of this conclusion, the disease-free equilibrium point of the pneumonia and meningitis coinfection model (1) is globally asymptotically stable if  *ℛ*_*eff*_ = max{ *ℛ*_1_, *ℛ*_2_} < 1.

### 2.10. Endemic Equilibrium Point and Its Stability

The endemic equilibrium point of the dynamical system (1) is obtained by making the right side of the system equal to zero providing that  *M*_*I*_ ≠ 0,  *P*_*I*_ ≠ 0 and *MP*_*I*_ ≠ 0. We have supposed the endemic equilibrium point of the model is denoted by  *E*_*pm*_^∗^ = (*S*^∗^, *M*_*v*_^∗^, *P*_*v*_^∗^, *MP*_*v*_^∗^, *M*_*I*_^∗^, *P*_*I*_^∗^, *MP*_*I*_^∗^, T^∗^, R^∗^) and the corresponding forces of infection are

(44) $$\begin{array}{c} {\alpha_{1}}^{*}=a\left({M_{I}}^{*}+{ℯ}_{1}{{MP}_{I}}^{*}\right)\text{ and }{\alpha_{2}}^{*}=b\left({P_{I}}^{*}+{ℯ}_{2}{{MP}_{I}}^{*}\right),\\ S^{*}=\frac{1}{\left({\alpha_{1}}^{*}+{\alpha_{2}}^{*}+\mu \right)}\left(\left(1-\pi \right)\lambda +\frac{\phi \rho \pi \lambda }{\left(\mu +\phi +\varepsilon_{2}\right)}+\frac{\left(1-\rho \right)\varphi \pi \lambda }{\left(\mu +\varphi +\varepsilon_{1}\right)}+Y\frac{\beta {\text{T}}^{*}}{\left(Y+\mu \right)}\right),\\ {M_{v}}^{*}=\frac{\left(1-\rho \right)\pi \lambda }{\left(\mu +\varphi +\varepsilon_{1}\right)},\\ {P_{v}}^{*}=\frac{\rho \pi \lambda }{\left(\mu +\phi +\varepsilon_{2}\right)},\\ {{MP}_{v}}^{*}=\left(\frac{\varepsilon_{1}}{\mu }\right)\left(\frac{\left(1-\rho \right)\pi \lambda }{\left(\mu +\varphi +\varepsilon_{1}\right)}\right)+\left(\frac{\varepsilon_{2}}{\mu }\right)\left(\frac{\rho \pi \lambda }{\left(\mu +\phi +\varepsilon_{2}\right)}\right),\\ {M_{I}}^{*}=\left(\frac{\alpha_{1}}{\left(\;\omega_{2}{\alpha_{2}}^{*}+\tau_{1}+\delta_{1}+\mu \right)}\right)\left(\frac{1}{\left({\alpha_{1}}^{*}+{\alpha_{2}}^{*}+\mu \right)}\left(\left(1-\pi \right)\lambda +\frac{\phi \rho \pi \lambda }{\left(\mu +\phi +\varepsilon_{2}\right)}+\frac{\left(1-\rho \right)\varphi \pi \lambda }{\left(\mu +\varphi +\varepsilon_{1}\right)}+Y\frac{\beta {\text{T}}^{*}}{\left(Y+\mu \right)}\right)\right),\\ {P_{I}}^{*}=\left(\frac{\alpha_{2}}{\left(\;\omega_{1}{\alpha_{1}}^{*}+\tau_{2}+\delta_{2}+\mu \right)}\right)\left(\frac{1}{\left(\alpha_{1}+{\alpha_{2}}^{*}+\mu \right)}\left(\left(1-\pi \right)\lambda +\frac{\phi \rho \pi \lambda }{\left(\mu +\phi +\varepsilon_{2}\right)}+\frac{\left(1-\rho \right)\varphi \pi \lambda }{\left(\mu +\varphi +\varepsilon_{1}\right)}+Y\frac{\beta {\text{T}}^{*}}{\left(Y+\mu \right)}\right)\right),\\ {{MP}_{I}}^{*}=\left(\frac{1}{\left(\tau_{3}+\mu \right)}\right)\left(\;\omega_{1}{\alpha_{1}}^{*}\right)\left(\frac{\alpha_{2}}{\left(\;\omega_{1}{\alpha_{1}}^{*}+\tau_{2}+\delta_{2}+\mu \right)}\right)\left(\frac{1}{\left({\alpha_{1}}^{*}+{\alpha_{2}}^{*}+\mu \right)}\left(\left(1-\pi \right)\lambda +\frac{\phi \rho \pi \lambda }{\left(\mu +\phi +\varepsilon_{2}\right)}+\frac{\left(1-\rho \right)\varphi \pi \lambda }{\left(\mu +\varphi +\varepsilon_{1}\right)}+Y\frac{\beta {\text{T}}^{*}}{\left(Y+\mu \right)}\right)\right)+\left(\left(\frac{\alpha_{1}\;\omega_{2}{\alpha_{2}}^{*}}{\left(\;\omega_{2}{\alpha_{1}}^{*}+\tau_{1}+\delta_{1}+\mu \right)\left({\alpha_{1}}^{*}+{\alpha_{2}}^{*}+\mu \right)\left(\tau_{3}+\mu \right)}\right)\left(\left(1-\pi \right)\lambda +\frac{\phi \rho \pi \lambda }{\left(\mu +\phi +\varepsilon_{2}\right)}+\frac{\left(1-\rho \right)\varphi \pi \lambda }{\left(\mu +\varphi +\varepsilon_{1}\right)}+Y\frac{\beta {\text{T}}^{*}}{\left(Y+\mu \right)}\right)\;\right),\\ {\text{T}}^{*}=\frac{\tau_{1}{M_{I}}^{*}+\tau_{2}{P_{I}}^{*}+\tau_{3}{{MP}_{I}}^{*}}{\left(\beta +\mu \right)},{\text{R}}^{*}=\frac{\beta {\text{T}}^{*}}{\left(Y+\mu \right)}. \end{array}$$

**Theorem 12 .**

The article "Appraisal and Simulation on Codynamics of Pneumonia and Meningitis with Vaccination Intervention: From a Mathematical Model Perspective" was published in 2022. Journal: Comput Math Methods Med.

The endemic equilibrium point  *E*_*pm*_^∗^  is locally asymptotically stable if the *ℛ*_*eff*_ > 1, otherwise it is unstable.

Proof: the local stability of the endemic equilibrium point of the full model is verified by using a numerical simulation in Section 4Figure 3.

## 3. Sensitivity Analysis and Numerical Simulations

In this section, we have carried out the sensitivity analysis to find the possible sensitive parameters having important implications to prevent and control the meningitis and pneumonia coinfection spread and the numerical simulations of model parameters and model solutions to approve the analytical results that we have done in Section 3.

In the numerical simulation of the meningitis and pneumonia coinfection model, we assessed the possible impact of controlling strategies on the dynamics of the disease.

### 3.1. Sensitivity Analysis

*Definition*. the normalized forward sensitivity index of a variable meningitis and pneumonia reproduction number denoted by the symbol  *ℛ*_*eff*_  that depends differentially on a parameter *ξ* is defined as SI(*p*) = *∂ℛ*_*eff*_/*∂ξ*∗*ξ*/*ℛ*_*eff*_ [2, 17].

Conducting sensitivity analysis provides a number of benefits for decision-makers. First, it acts as an in-depth study of all the variables. Secondly, it allows decision-makers to identify where they can make improvements in the future. In our case, it helps us to determine the relative and importance of different parameters in meningitis and pneumonia incidence and prevalence. The most sensitive parameter has the magnitude of the sensitivity index larger than that of all other parameters. We have manipulated the sensitivity index in terms of

(45) $$\begin{array}{c} \;R_{eff}=\max\left\{\frac{a\lambda \left(1-\pi \right)}{\left(\;\tau_{1}+\delta_{1}+\mu \right)\mu }+\frac{\phi \rho \left(\mu +\varphi +\varepsilon_{1}\right)+\varphi \left(1-\rho \right)\left(\mu +\phi +\varepsilon_{2}\right)}{\left(\mu +\phi +\varepsilon_{2}\right)\mu }\left(\frac{\pi \lambda a}{\tau_{1}+\delta_{1}+\mu }\right),\frac{b\lambda \left(1-\pi \right)}{\left(\;\tau_{2}+\delta_{2}+\mu \right)\mu }+\frac{\phi \rho \left(\mu +\varphi +\varepsilon_{1}\right)+\varphi \left(1-\rho \right)\left(\mu +\phi +\varepsilon_{2}\right)}{\left(\mu +\phi +\varepsilon_{2}\right)\mu }\left(\frac{\pi \lambda b}{\tau_{2}+\delta_{2}+\mu }\right)\right\}. \end{array}$$

We could have manipulated the sensitivity index in terms of *ℛ*_1_ and *ℛ*_2_ since *ℛ*_*eff*_ = max{*ℛ*_1_, *ℛ*_2_}.

Sensitivity analysis results and the numerical simulation are given in this section with parameter values given in Table 2 with the initial population of the full meningitis and pneumonia coinfection model.

The article "Appraisal and Simulation on Codynamics of Pneumonia and Meningitis with Vaccination Intervention: From a Mathematical Model Perspective" was published in 2022. Journal: Comput Math Methods Med.

#### 3.1.1. The Sensitivity Indices for *ℛ*_1_

In this section, we have stated the sensitivity indices for  *ℛ*_1_. Using the values of the parameters in Table 2, the sensitivity indices for *ℛ*_1_ is calculated in the following:

1. SI(*a*) = *∂ℛ*_1_/*∂a*∗(*a*/*ℛ*_1_)(*∂ℛ*_1_/*∂a*) = *λ*[1 − *π*]/*μ*(*μ* + *δ*_1_ + *τ*_1_) + (*πλ*(*ϕρ*[1 + *μ* + *φ*] + (1 + *μ* + *ϕ*)*φ*[1 − *ρ*]))/*μ*(1 + *μ* + *ϕ*)(*μ* + *δ*_1_ + *τ*_1_)⇒*SI*(*a*) = 1
2. SI(*δ*_1_) = *∂ℛ*_1_/*∂δ*_1_∗*δ*_1_/*ℛ*_1_ ⇒ *∂ℛ*_1_/*∂δ*_1_ = −*aλ*[1 − *π*]/*μ*(*μ* + *δ*_1_ + *τ*_1_)^2^ − (*aπλ*(*ϕρ*[1 + *μ* + *φ*] + (1 + *μ* + *ϕ*)*φ*[1 − *ρ*]))/*μ*(1 + *μ* + *ϕ*)(*μ* + *δ*_1_ + *τ*_1_)^2^⇒*SI*(*δ*_1_) = −*δ*_1_/(*μ* + *δ*_1_ + *τ*_1_)

Following the procedures we have generalized and stated the sensitivity parameters as follows:

In this section, the obtained figure was explored with parameter values given in Table 2, and we have gotten *ℛ*_1_ = 12.33 at *a* = 0.9, which implies meningitis has been expanded throughout the considered community, and additionally, we have manipulated the sensitivity indices for other parameters as show in Figure 4. The obtained sensitivity analysis shows that the recruitment rate *λ* and meningitis effective contact rate *a* have the highest impact on *ℛ*_1_.

#### 3.1.2. The Sensitivity Indices for *ℛ*_2_

In this section we have presented the sensitivity indices for  *ℛ*_2_ . Using the values of parameters in Table 2, the sensitivity indices for *ℛ*_2_ is calculated in following chart.

1. SI(b) = *∂ℛ*_2_/*∂*b∗(b/*ℛ*_2_)(*∂ℛ*_2_/*∂b*) = (*πλϕρ*[1 + *μ* + *φ*] + (1 + *μ* + *ϕ*)(*λ*[1 − *π*] + *πλφ*[1 − *ρ*]))/*μ*(1 + *μ* + *ϕ*)(*μ* + *δ*_2_ + *τ*_2_)⇒*SI*(*b*) = 1
2. *SI*(*δ*_2_) = *∂ℛ*_2_/*∂δ*_2_∗*δ*_2_/*ℛ*_2_⇒*∂ℛ*_2_/*∂δ*_2_ = (*b*(*πλ*((1 + *μ*)*ρ*(*ϕ* − *φ*) + (1 + *μ* + *ϕ*)*φ*) + (1 + *μ* + *ϕ*)*λ*[1 − *π*]))/*μ*(1 + *μ* + *ϕ*)(*μ* + *δ*_2_ + *τ*_2_)

Following the procedures we have generalized and stated the sensitivity parameters as follow

In this section, the obtained figure was explored with parameters values given in Table 2 and we have got *ℛ*_2_ = 15.1 at *b* = 0.85 which implies pneumonia has been expanded throughout the considered community and additionally we have manipulated the sensitivity indices for another parameters as show in Figure 2 above. The obtained sensitivity analysis shows that the recruitment rate *λ* and pneumonia effective contact rate *b* have the highest impact on *ℛ*_2_.

### 3.2. Numerical Simulations

MATAB software is used to ensure the accuracy of the mathematical terminology descriptions and the validity of the analytical solution. To show the verification of the analytical solution we acquired in the previous part, we utilized the MATLAB code ODE 45. Additionally, we have shown and investigated the effects of a number of traits (parameters) that are related to meningitis and pneumonia coinfection illness.

The article "Appraisal and Simulation on Codynamics of Pneumonia and Meningitis with Vaccination Intervention: From a Mathematical Model Perspective" was published in 2022. Journal: Comput Math Methods Med.

#### 3.2.1. Local Stability of the Endemic Equilibrium Point

The parameters from Table 2 were used to run a numerical simulation using the ODE 45, which produced the results shown in Figure 3. From Figure 3, we can observe that after a year, the solutions of the meningitis and pneumonia coinfection dynamical system (1) will be approaching to the endemic equilibrium point of the meningitis and pneumonia coinfection depends on the value of *ℛ*_*eff*_ = max{ *ℛ*_1_, *ℛ*_2_}. More specifically, Figure 3 shows that after a time, the solutions of the meningitis and pneumonia infection transmission dynamics will be converging to its endemic equilibrium point, i.e., the endemic equilibrium point is locally asymptotically stable whenever *a* = 0.9 and  *ℛ*_*eff*_ = max {*ℛ*_1_, *ℛ*_2_} = 15.1 > 1. This mathematical conclusion illustrates the physical phenomena known as the proliferation and spread of meningitis and pneumonia coinfection regularly happening throughout the population which is confined to a certain location.

Figure 5 demonstrates that while the  *ℛ*_*eff*_ = max{ *ℛ*_1_, *ℛ*_2_} < 1, the solution of the system is converged to the disease-free equilibrium point.

#### 3.2.2. The Impact of Meningitis Treatment Rate on Meningitis and Pneumonia Coinfected Populations

We looked at how the coinfected class was affected by  *τ*_3_ in this part. We can see from Figure 6 that the prevalence of meningitis and pneumonia coinfection decreases as values of  *τ*_3_ rise. To manage the disease in the community, public authorities must focus on increasing the values of the treatment rate *τ*_3_.

#### 3.2.3. The Impact of Meningitis Treatment Rate on Coinfected Class

The endeavor we conducted about the impact of  *τ*_1_ on the coinfected class is illustrated in Figure 7. The figure shows that the population with coinfections of meningitis and pneumonia is decreasing as the values of the meningitis treatment rate, indicated by  *τ*_1_, rise. The most crucial thing to remember is that treating just meningitis-infected people can significantly reduce the cooccurrence of meningitis and pneumonia infections in communities, which is one of the study's main findings.

As a result, we advise the stakeholders to maximize the meningitis treatment rate in order to confine and stop the spread of the meningitis and pneumonia coinfection illness in the community.

The article "Appraisal and Simulation on Codynamics of Pneumonia and Meningitis with Vaccination Intervention: From a Mathematical Model Perspective" was published in 2022. Journal: Comput Math Methods Med.

#### 3.2.4. The Impact of Pneumonia Treatment Rate on Coinfected Class

The influence of pneumonia treatment rate (*τ*_2_) on the coinfected class is shown in Figure 8.

The graph shows that when the incidence of pneumonia treatment rises, the population with coinfections of meningitis and pneumonia declines. This study's other key observation is that treating pneumonia-infected people only has a substantial impact on reducing the cooccurrence of meningitis and pneumonia infections in communities, which is perhaps most relevant. In order to prevent and slow the spread of the meningitis and pneumonia coinfection illness in the community, we advise the stakeholders to maximize the values of the pneumonia treatment rate of *τ*_2_.

#### 3.2.5. The Impact of Parameters on  *ℛ*_*eff*_ = max{ *ℛ*_1_, *ℛ*_2_}

In this subsection, as we see in Figure 9, we have investigated the effect of vaccination (*ε*_2_) and the effective reproduction number *ℛ*_*eff*_ = max{ *ℛ*_1_, *ℛ*_2_}. The figure reflects that when the value of *ε*_2_ increases, both  *ℛ*_1_  and *ℛ*_2_ decrease, which implies that the maximum of them also declines.

Moreover, the value  *ℛ*_*eff*_ = max{ *ℛ*_1_, *ℛ*_2_}  becomes smaller than one when the value of *ε*_2_ > 0.39.

In this subsection, as we can see in Figure 10, we have investigated the effect of vaccination (*ε*_1_) and the effective reproduction number *ℛ*_*eff*_ = max{ *ℛ*_1_, *ℛ*_2_}. The figure reflects that when the value of  *ε*_1_ increases, both  *ℛ*_1_ and  *ℛ*_2_ decrease, which implies that the maximum of them also declines.

Moreover, the value  *ℛ*_*eff*_ = max{ *ℛ*_1_, *ℛ*_2_}  becomes smaller than one when the value of  *ε*_1_ > 0.258.

Figure 11 elaborates the investigation of effect contact rates *a* and *b* on  *ℛ*_*eff*_ = max{ *ℛ*_1_, *ℛ*_2_}.The figure represents that as the values of *a* and *b* increase, both  *ℛ*_1_ and  *ℛ*_2_ increase. To have the minimum values of  *ℛ*_*eff*_ = max{ *ℛ*_1_, *ℛ*_2_}, the value of *a* and *b* should be less than 0.19. As a result, we urge all relevant parties to pay close attention to the effectiveness of the pneumonia vaccine in preventing the coinfection of meningitis and pneumonia in society.

In this subsection, as we see in Figure 12, we have investigated the effect of a portion of vaccination of pneumonia protection portion *ρ* on the effective reproduction number  *ℛ*_*eff*_ = max{*ℛ*_1_, *ℛ*_2_}. The figure reflects that when the value of *ρ* increases, both  *ℛ*_1_ and  *ℛ*_2_ decrease, which implies that the maximum of them also declines. Moreover, when the value of *ρ* > 0.629, the value of  *ℛ*_2_  is less than one; when the value of  *ρ* > 0.831, the value of  *ℛ*_1_ is less than one.

The article "Appraisal and Simulation on Codynamics of Pneumonia and Meningitis with Vaccination Intervention: From a Mathematical Model Perspective" was published in 2022. Journal: Comput Math Methods Med.

This suggests that if and only if the percentage of pneumonia vaccination rate is higher than 0.831, then  *ℛ*_*eff*_ = max{ *ℛ*_1_, *ℛ*_2_} < 1. Therefore, to avoid and regulate the dynamic transmission of meningitis and pneumonia coinfection, public authorities must look to increase the gains of the pneumonia vaccination portion.

Figure 13 elaborates the investigation of the effect of pneumonia vaccination wanes (*ϕ*) on  *ℛ*_*eff*_ = max{ *ℛ*_1_, *ℛ*_2_}.The figure represents as the value of *ϕ* increases, both  *ℛ*_1_  and *ℛ*_2_ increase. To have the minimum values of  *ℛ*_*eff*_ = max{ *ℛ*_1_, *ℛ*_2_}, the value *ϕ* should be less than 0.4. As a result, we urge all relevant parties to pay close attention to the effectiveness of the pneumonia vaccine in preventing the coinfection of meningitis and pneumonia in society.

Figure 14 explains the investigation of the effect of meningitis vaccination wanes (*φ*) on *ℛ*_*eff*_ = max{ *ℛ*_1_, *ℛ*_2_}. The graph illustrates how both  *ℛ*_1_ and  *ℛ*_2_  grow when the value of *φ* rises. Our conclusion from this finding is that when the value of *φ* is smaller than 0.396, the minimal value of *ℛ*_*eff*_ = max{ *ℛ*_1_, *ℛ*_2_} is reached. The effectiveness of the meningitis vaccination in avoiding the coinfection of meningitis and pneumonia in society should thus be closely monitored, thus we encourage all pertinent parties to pay attention for it.

Analytic solution of some differential equations is complicated and tough. In such case, we need a numerical simulation of the system. In our case we have used a numerical simulation for stability analysis of steady state and obtained the result; after a year, the solutions of the meningitis and pneumonia coinfection dynamical system will tend to the endemic equilibrium point of the model. This expression of the plot illustrates the biological meaning of the proliferation and spread of meningitis and pneumonia coinfection which is regularly happening throughout the population of which is confined to a certain location. Additionally, we have used a numerical simulation to investigate the effects of a number of traits (parameters) that are related to the meningitis and pneumonia coinfection illness, such as, treatment rate, meningitis treatment rate, pneumonia treatment rate, effect of vaccination, and effective contact rate and vaccination wanes rate. As a result, we have shown that increasing availability to meningitis and pneumonia prevention, treatment, and meningitis and pneumonia coinfection vaccine has a significant influence on the frequency of meningitis and pneumonia in a particular population.

The article "Appraisal and Simulation on Codynamics of Pneumonia and Meningitis with Vaccination Intervention: From a Mathematical Model Perspective" was published in 2022. Journal: Comput Math Methods Med.

## 4. Discussion

We addressed the epidemiology and historical context of meningitis and pneumonia in Section 1.

In Section 2, the deterministic meningitis and pneumonia coinfection dynamical system was built by dividing the entire human population into nine groups based on the severity of the infection. Moreover, we looked at the model's descriptive phenomena, including the model's prospective solutions being positive, the dynamical system being bounded, the existence of a disease-free equilibrium point, the existence of an effective reproduction number using the next generation matrix technique, the existence of endemic equilibriums, and the stability analysis of the disease-free equilibrium point using the Routh-Hurwitz criteria in this section. Additionally, the Routh-Hurwitz criteria were used to demonstrate the local stability of endemic equilibrium points of submodels, and we were able to conclude that these points are locally asymptotically stable if the reproduction number is less than one. Nevertheless, the endemic equilibrium point of the combined meningitis and pneumonia coinfection model is revealed by numerical simulation presented in Section 3 by Figure 3, i.e., the endemic equilibrium point is locally asymptotically stable just when  *a* = 0.9,  *b* = 0.85, and *ℛ*_*eff*_ = max{*ℛ*_1_ = 12.33, *ℛ*_2_ = 15.1} > 1.

Through the use of numerical simulation, we have examined the effects of several parameters on the effective reproduction rate as well as the prevention and control of the development of meningitis and pneumonia infections in Section 3. The results show that increasing availability to meningitis and pneumonia prevention, treatment, and meningitis and pneumonia coinfection vaccine has a significant influence on the frequency of meningitis and pneumonia in a particular population. The optimal control analysis of pneumonia and meningitis coinfection [8] having solely evaluated prevention for both meningitis and pneumonia, we found that preventative regulation had a significant influence on reducing the spread of meningitis, pneumonia, and their coinfection within the given time frame. Efforts to avoid pneumonia and treat meningitis are two more techniques addressed in this study. They discovered that each of the stated measures is successful in reducing the growth of the infectious populations that only have meningitis, pneumonia, or both throughout the allotted time frame.

A mathematical model of seven nonlinear differential equations for the pneumonia and meningitis coinfection with PCV vaccination for a newly born population and treatment for coinfected class has also been developed and entitled as “mathematical model analysis and numerical simulation for codynamics of meningitis and pneumonia infection with intervention” [5]. They have taken into account the PCV13 (pneumococcal conjugate vaccine), which is a vaccination given to infants and protects against a variety of pneumococcal bacteria that can cause the most severe forms of pneumococcal illness, such as pneumonia and meningitis. Additionally, researchers [7] have demonstrated that the availability of hospital beds, medicines, and other treatment options all contribute to a decline in the number of cases of bacterial meningitis. However, they observe that an increased recruitment rate causes a backward split in a town with few hospital beds.

The article "Appraisal and Simulation on Codynamics of Pneumonia and Meningitis with Vaccination Intervention: From a Mathematical Model Perspective" was published in 2022. Journal: Comput Math Methods Med.

Finally, they advise using vaccination when there is a large influx of new people. Numerous studies have demonstrated that meningitis and pneumonia infections may be wiped out in the community when treatment and immunization efforts are combined. Despite treatment interventions, these diseases and their combined forms continue to exist in the entire population. Three different vaccine combinations with similar treatments were not taken into account in any model across all studies. In contrast to the previous studies described above, the model developed in this study took into consideration all three vaccines, namely the meningitis vaccine, the pneumonia vaccine, and people who had received both the vaccine and therapy at the same time.

## 5. Conclusion

The study is aimed at building and examining a compartmental deterministic mathematical model of the dynamics of the spread of the coinfection of meningitis and pneumonia. In the population under the study, this model considered how vaccination and therapy of single infection of meningitis or pneumonia may reduce the risk of meningitis and pneumonia coinfection. When the effective reproduction number is smaller than unity, the model possesses a disease-free equilibrium point that is locally asymptotically stable. The outcome of the numerical simulation demonstrates that when  *ℛ*_*eff*_ > 1, the meningitis and pneumonia coinfection model's endemic equilibrium point is locally asymptotically stable.

Besides obtaining the model's matching effective reproduction number  *ℛ*_*eff*_, we were able to identify the effects of changing specific parameter values and provide future guidance for the public's partners. Our findings have significant public health implications because they affect whether a disease is eradicated or persists in the community under investigation.

As a result of our numerical findings which show that *ℛ*_*eff*_ = 15.1 at *b* = 0.85 and *a* = 0.9, we notify public authorities to focus on raising or maximizing the values of the involved individuals' meningitis vaccination, pneumonia vaccination, and meningitis and pneumonia coinfection vaccination as well as treatment rates in order to reduce and eradicate the disease from the study's target community. Finally, other key results of this study are meningitis contact rates, pneumonia contact rates, and vaccination deficits of corresponding diseases that have contributed immensely to the spread of meningitis and pneumonia coinfection in the community.

The article "Appraisal and Simulation on Codynamics of Pneumonia and Meningitis with Vaccination Intervention: From a Mathematical Model Perspective" was published in 2022. Journal: Comput Math Methods Med.

## Figures and Tables

**Figure 1:** Schematic diagram of full pneumonia and meningitis codynamics.

**Figure 2:** Sensitivity indices for *ℛ*_2_.

**Figure 3:** Stability of endemic equilibrium when  *ℛ*_*eff*_ = max{ *ℛ*_1_, *ℛ*_2_}>1.

**Figure 4:** Sensitivity indices for *ℛ*_1_.

**Figure 5:** model representation when  *ℛ*_*eff*_ = max{ *ℛ*_1_, *ℛ*_2_}  <1

**Figure 6:** The effect of treatment rate on the coinfected population.

**Figure 7:** Plot effect of meningitis treatment rate on the coinfected groups.

**Figure 8:** Plot effect of pneumonia treatment rate on the coinfected class.

**Figure 9:** Effect of vaccination (*ε*_2_) on reproduction numbers.

**Figure 10:** Effect of vaccination (*ε*_1_) on reproduction numbers.

**Figure 11:** Effect of effective contact rate on reproduction numbers.

**Figure 12:** Effect of a portion of pneumonia vaccination on reproduction numbers.

**Figure 13:** Effect of pneumonia vaccination wanes rate on reproduction numbers.

**Figure 14:** Effect of meningitis vaccination wanes rate on reproduction numbers.

**Table 1:** Descriptions of parameters of the model.

Parameter	Description
*a*	Meningitis effective contact rate
*b*	Pneumonia effective contact rate
*τ*_1_	The rate at which meningitis-infected individuals are treated enter to and treated class
*τ*_2_	The rate at which pneumonia-infected individuals are treated and enter to treated class
*τ*_3_	The rate at which meningitis and pneumonia coinfected individuals are treated and enter to treated class
*β*	The rate at which treated class recovered
*μ*	Natural death rate
*δ*_1_	Meningitis-only caused death rate
*δ*_2_	Pneumonia-only caused death rate
*δ*_3_	Meningitis and pneumonia coinfection caused death rate.
*ω*_1_	Modification parameter and *ω*_1_ ≥ 1
*ω*_2_	The modification parameter and *ω*_2_ ≥ 1
*Y*	Rate of loss of immunity
*π*	The portion of vaccinated new born
*λ*	Recruitment rate
*ε*_2_	The rate at which a pneumonia vaccinated individual takes meningitis vaccination
*ε*_1_	The rate at which a meningitis vaccinated individual takes pneumonia vaccination
*ϕ*	Pneumonia vaccine wanes rate
*φ*	Meningitis vaccine wanes rate
*ρ*	The portion in which pneumonia vaccine is given

The article "Appraisal and Simulation on Codynamics of Pneumonia and Meningitis with Vaccination Intervention: From a Mathematical Model Perspective" was published in 2022. Journal: Comput Math Methods Med.

**Table 2:** Parameter values used for the coinfection model simulation.

Parameter	Values	Unit	Source
*a*	0.9	size^−1^∗Time^−1^	[8]
*b*	0.007-0.6	size^−1^∗Time^−1^	[8]
*τ*_1_	0.02	Time^−1^	[8]
*τ*_2_	0.012	Time^−1^	[8]
*τ*_3_	0.31	Time^−1^	[8]
*β*	0.06 -0.13	Time^−1^	[16, 17]
*μ*	0.01	Time^−1^	[8]
*δ*_1_	0.002-0.2	Time^−1^	[8]
*δ*_2_	0.006-05	Time^−1^	[8]
*δ*_3_	0.008-0.7	Time^−1^	[8]
*ω*_1_	1	Time^−1^	Assumed
*ω*_2_	1	Time^−1^	Assumed
*Y*	**0.007-0.4**	Time^−1^	[8]
*π*	0.105	Time^−1^	[8]
*λ*	**0.0413** ^∗^ *N*_0_	Size∗Time^−1^	[8]
*ε*_2_	0.007	Time^−1^	Assumed
*ε*_1_	0.025	Time^−1^	Assumed
*ϕ*	0.0115	Time^−1^	[22]
*φ*	0.5	Time^−1^	[23]
*ρ*	0.05	Time^−1^	[21]

## Data Availability

Data used to support the findings of this study are included in the article
